The article "Computation of differential and integral operators using ℳ-polynomials of gold crystal" was retracted in 2025. Reasons: plagiarism; unreliable results or conclusions; concerns about the peer review; concerns about the citations.

# Computation of differential and integral operators using M-polynomials of gold crystal

**DOI:** 10.1016/j.heliyon.2024.e34419

**Published:** 2024-07-14

**Authors:** Abdul Rauf Khan, Saad Amin Bhatti, Muhammad Imran, Ferdous M.O. Tawfiq, Murat Cancan, Shahid Hussain

**Affiliations:** a Department of Mathematics, Faculty of Sciences, Ghazi University, Dera Ghazi Khan, 32200, Pakistan; b Department of Mathematical Sciences, United Arab Emirates University, Al Ain, 15551, United Arab Emirates; c Mathematics Department, College of Science, King Saud University, Riyadh 11495, 22452, Saudi Arabia; d Faculty of Education, Yuzuncu Yil University, Van, Turkey; e Energy Engineering Division, Department of Engineering Science and Mathematics, Lulea University of Technology, Lulea, 97187, Sweden

**Keywords:** Gold Crystal, Molecular structure, M-Polynomial, Topological indices, Differential operators, Integral operators, Computation

## Abstract

Gold is generally considered a noble metal since it is inherently inert in its bulk state. However, gold demonstrates reactivity when it is in its ionic state. The inherent inertness of bulk gold has resulted in its widespread recognition as a vital raw material in various biomedical processes. The applications of these technologies include drug delivery microchips, dental prostheses, reconstructive surgery, culinary additives, and cardiovascular stents. Gold can also exist in molecules or ions, particularly gold ions, which facilitates the production of gold nanomaterials. In this paper, we have computed differential and integral operators by using the M-Polynomial of gold crystals and by utilizing this polynomial, we have also computed eleven topological indices like $1^{st}$ Zagreb, $2^{nd}$ Zagreb, Hyper, Sigma, Second Modified, General Randic, General Reciprocal Randic, $3^{rd}$ Redefined Zagreb, Symmetric Division Degree, Harmonic, Inverse Sum indices for the structure of Gold crystal.

## 1 Introduction

The presence of emergent features at a larger scale makes the multiscale morphologies of substances and devices composed of multiple nanosized components examples of complex structures [1], [2], [3]. Exerting control over the structure of a nanomaterial would yield remarkable transformations and establish a firm basis for its utilization in nanotechnology. Nevertheless, the unique properties of nano-structured systems and the increased fluctuations at the nanoscale present valuable obstacles for theoretical and computational modelling [4], necessitating an advancement beyond existing methodologies [5]. Using graph theory methodologies and accurate alignment with mathematical graphs (networks) has significantly propelled the advancement of modelling intricate structures in recent times. The primary concept is to discern the constituents of the graphs, namely the nodes and the edges (hyperlinks) that connect the nodes, while considering the limitations imposed by the system's characteristics. Within a network that represents a complex system, it is common for both nodes and edges to generate extra properties that need to be considered [6].

The article "Computation of differential and integral operators using ℳ-polynomials of gold crystal" was retracted in 2025. Reasons: plagiarism; unreliable results or conclusions; concerns about the peer review; concerns about the citations.

The discovery of new types of graphs raises the necessity for sound, difficult mathematical concepts. Consequently, complex networks create a new division of science and technology [7]. As a result, the measurement-capable exploration of the fundamental complex systems is made possible by employing graph theory techniques [8], [9]. In particular, those procedures significantly advanced the fields of bioinformatics [10] and tectonophysics [11] and increased the quantitative analysis of social structures [12]. The complex network principle has recently been used to study a wide range of nanoscale system-related issues.

Topological indices are numerical values calculated from the molecular graph of a chemical substance and they maintain their value even when the graph is rearranged. A degree-based topological index is a type of index that is determined by the degrees of the molecular graph [13], [14]. It belongs to a family of indices that can be utilized to highlight and simulate specific characteristics of chemical compounds [15], [16].

Topological indices are numerical representations of the structure of molecules and are employed in the development of qualitative structure-activity relationships (QSARs) [17], [18]. Degree-based topological indices are the most widely recognized invariants in such categories [19], [20]. The mathematical calculations show how the structure relates to many physical characteristics, chemical reactivity, and biological activity [21]. The study focuses on the utilization of topological indices to analyze the chemical structures and QSPR/QSAR analysis of antiviral medicines under investigation for the treatment of COVID-19 patients [22]. The interrelation between a molecule's graphical structure and other qualities such as heat of formation, boiling temperature, strain energy, stiffness, and fracture toughness is widely acknowledged [23], [24].

Topological indices generally refer to numerical quantities or parameters that are calculated based on the topology of a molecular or crystal structure [25], [26]. Topological indices are numbers or parameters obtained from a chemical structure's graph theory representation [27]. Without deliberately considering the spatial arrangement of atoms in three-dimensional space, they are used in chemistry and molecular modelling to measure numerous molecular features, such as size, shape, branching, connectivity, and electrical structure [28]. The foundation for topological indices is transforming a molecular graph into an index that describes the topology of that network [29]. Molecular modelling is used to study the structure, characteristics, and activity of chemical molecules related to one another. Molecular descriptors played a key role in learning the main chemical structure topics, such as chemistry [30], [31], pharmacology [32] etc. Topological indices were revealed to be one of the most important molecular descriptors in the (QSAR)/(QSPR) investigation [33].

The article "Computation of differential and integral operators using ℳ-polynomials of gold crystal" was retracted in 2025. Reasons: plagiarism; unreliable results or conclusions; concerns about the peer review; concerns about the citations.

Rashid et al. centre their attention on a category of smart polymers that find widespread application in the development of anticancer medications [34]. Hayat et al. studied valency-based chemical network topological indices. Using real information, they carried out precise comparative studies to examine the effectiveness of a few valency-based indices in practice [35] and Khan et al. examined bladder cancer drugs in [36]. Using a polynomial technique, Mondal et al. assessed several degree-based and neighbourhood degree sum-based topological indices for antiviral medications [37] and metrics, topological indices, and edge metric resolvability are determined by Sharma et al. in [38]. The $E_{v}$ and $V_{e}$-degree-based topological indices for the generalized carbon nanocones, CNCr[s], are discussed by Sharma et al. [39] and examined the three important benzenoid classes in [40]. Manzoor et al. investigated the crystallographic structure of cuprite and the chemical graph of titanium difluoride's crystal structure. They then estimated the entropies of these structures by establishing a relationship between degree-based topological indices [41] and Gao et al. investigated M-Polynomials in [42]. CCS[m], one of the valuable carbon allotropes, is one of the degree-based multiplicative topological indices of the cubic carbon crystalline structure for levels m = 3–10, as determined by Sharma et al. [43]. The hyper-Zagreb coindex and polynomials of specific benzenoid structures were presented by Sharma et al. in [44].

Hosoya polynomial and Wiener polynomial board play a crucial role in distance-based topological indices. The Hosoya polynomial allows for the straightforward assessment of a wide range of distance-based indices. Deutsch and Klavzar recently achieved a comparable innovation within the context of degree-based indices [45]. In 2014, Deutsch and Klavzar introduced the concept of the M-Polynomial, which serves as an analogue to the Hosoya polynomial. This polynomial is used to determine the closed form of various degree-based topological indices [46], [47]. In the same context, the M-Polynomial serves as a relevant measure. It allows us to obtain closed-form expressions for degree-based topological indices [48], [49], [50], [51], [52], [53], [54]. Several recent works focus on identifying the M-Polynomial of a particular chemical graph. In the study by Raza et al. [55], two molecular graphs, namely $ND_{1}[2]$ and $ND_{2}[2]$, were analyzed. The authors calculated the M-Polynomials for both graphs and used them to determine certain degree-based topological indices for the chemical graphs.

The article "Computation of differential and integral operators using ℳ-polynomials of gold crystal" was retracted in 2025. Reasons: plagiarism; unreliable results or conclusions; concerns about the peer review; concerns about the citations.

Numerous areas of science and technology now use structure-based investigation of nanoparticles. Along with the more traditional uses for nanoparticles like catalysis and photography, nanoscale and aerosol studies have also become crucial. Due to its intriguing behaviour, including its quasi-melting [56] and minimal affinity for petrol absorption [57], gold has emerged as one of the most pertinent instances to examine in this context. These statistics make it possible to study the behaviour of metallic particles while minimizing the effects of air contamination. Due to the face-centred cubic crystal structure of gold, each unit cell contains four gold atoms. The volume of the unit cell in gold, whose lattice parameter is 4:08, is 0:0679 $nm^{3}$. Although the gold nanoparticles generally are almost spherical, their unit cells are cubic. We determine a unit cell's gold atom count from its crystal structure [57]. Bulk gold is face-centred cubic (fcc), and rare native gold crystals occasionally show extremely uniform cubic, octahedral, or rhombododecahedral crystal shapes consistent with the fcc geometry. This generalization applies to particles as tiny as 10 nm (with around 28,000 gold atoms), but it becomes more complicated for progressively lower sizes. Nanoparticles' structure and outward form between 1 and 10 nm are hotly contested topics [58]. The challenges of trying to describe such minute objects physically have intensified this argument. The structure of gold nanoparticles has been predicted by calculation in many different approaches. In general, neither the results of these computations nor those obtained through experimental methods are entirely consistent. Disputed assertions are made regarding icosahedral or decahedral shapes [59]. In [60], the author computed the $V_{e}$-degree, $E_{v}$-degree, and degree-based topological indices of fenofibrate. In 2023, the author computes some novel degree-based topological descriptors of Fenofibrate using M-Polynomial [61].

In this paper, we aim to compute the M-Polynomial of Gold Crystal and differential and integral operators of the computed M-Polynomial as shown in Fig. 1. We will also determine the first Zagreb M-Polynomial, second Zagreb M-Polynomial, and General Randic M-Polynomial. We also recover the first and second Zagreb indices, the Hyper Zagreb index, the Sigma index, the second Modified and Redefined third Zagreb index, the Symmetric Division index, the Harmonic index, the Randic and the General Randic indices and the Inverse Sum index by using the computed M-Polynomial of Gold crystal structure. For a more detailed study of the topological indices and their applications, we refer to the references [62], [63], [64], [65].

The article "Computation of differential and integral operators using ℳ-polynomials of gold crystal" was retracted in 2025. Reasons: plagiarism; unreliable results or conclusions; concerns about the peer review; concerns about the citations.

**Figure 1:** Structure of Gold Crystal.

The “Hosoya polynomials” were introduced in 1988 to refer to a certain form of polynomials. These polynomials are also known as M-Polynomials. These polynomials are related to the topological descriptors that are dependent on the valency of atoms. The M-Polynomials of a network can be utilized to determine the topological characteristics in a particular fashion. The variables *x* and *y* represent unknown quantities. The symbol $\rho_{\left(i,j\right)}$ denotes the number of edges in a graph, where d(τ) represents the degree of a vertex *τ*, which is the number of edges incident to that vertex. The term “degree of that vertex” refers to the degree of a specific vertex. The M-Polynomial is defined as follows: for any pair of indices *i* and *j* where i≤j, $\rho_{\left(i,j\right)}$ represents the number of edges in the graph G.

(1) $$M(G;x,y)=\sum_{i\leq j}\rho_{\left(i,j\right)}x^{i}y^{j}$$

The atom-based $1^{st}$ Zagreb index which depends on the valency-based topological descriptors is given as follows for the graph G

(2) $$M_{1}(G)=\sum_{\tau \sigma \in E(G)}(d(\tau )+d(\sigma ))$$

The $2^{nd}$ Zagreb index for the graph G is

(3) $$M_{2}(G)=\sum_{\tau \sigma \in E(G)}(d(\tau ).d(\sigma ))$$

The M-Polynomial of above mentioned first and second Zagreb index are

(4) $$M_{M_{1}}(G)=(D_{x}+D_{y})(M(G;x,y))$$

(5) $$M_{M_{2}}(G)=(D_{x}.D_{y})(M(G;x,y))$$

The General Randic index and its corresponding M-Polynomial are given as

(6) $$R_{\alpha }(G)=\sum_{\tau \sigma \in E(G)}{\left(d(\tau ).d(\sigma )\right)}^{\alpha }$$

(7) $$M_{R_{\alpha }}(G)=(D_{x}^{\alpha }D_{y}^{\alpha })(M(G;x,y))$$

The differential and integral operators are defined as below

(8) $$D_{x}=x\frac{\partial (M(G;x,y))}{\partial x}$$

(9) $$D_{y}=y\frac{\partial (M(G;x,y))}{\partial y}$$

(10) $$I_{x}=\int_{0}^{x}\frac{1}{z}(M(G;z,y))dz$$

(11) $$I_{y}=\int_{0}^{y}\frac{1}{z}(M(G;x,z))dz$$

The Edge Division of Gold Crystal is described below in Table 1.

The article "Computation of differential and integral operators using ℳ-polynomials of gold crystal" was retracted in 2025. Reasons: plagiarism; unreliable results or conclusions; concerns about the peer review; concerns about the citations.

**Table 1:** Edge Division of Gold Crystal.

(*d*(*τ*),*d*(*σ*))	Cardinality
(4,6)	24
(4,9)	20(r+s+t)-120
(4,13)	16(rs+st+rt)-64(r+s+t)+192
(4,18)	12rst-24(rs+st+rt)+48(r+s+t)-96
(6,9)	24
(9,9)	4(r+s+t)-36
(9,13)	8(r+s+t)-48
(13,13)	4(rs+st+rt)-20(r+s+t)+72
(13,18)	2(rs+st+rt)-8(r+s+t)+24
(18,18)	3rst-7(rs+st+rt)+16(r+s+t)-36

## 2 M-Polynomials of Gold Crystal

Theorem 1 *Let* GCR *be a graph of gold crystal and* M(GCR;x,y) *is the* M *-polynomial for* GCR(x,y)

$$M(\mathrm{GCR};x,y)=24x^{4}y^{6}+[20(r+s+t)-120]x^{4}y^{9}+[16(rs+st+rt)-64(r+s+t)+192]x^{4}y^{13}+[12rst-24(rs+st+rt)+48(r+s+t)-96]x^{4}y^{18}+24x^{6}y^{9}+[4(r+s+t)-36]x^{9}y^{9}+[8(r+s+t)-48]x^{9}y^{13}+[4(rs+st+rt)-20(r+s+t)+72]x^{13}y^{13}+[2(rs+st+rt)-8(r+s+t)+24]x^{13}y^{18}+[3rst-7(rs+st+rt)+16(r+s+t)-36]x^{18}y^{18}$$

Proof Let GCR be a graph of gold crystal. In view of Table 1 and Equation (1), we get the M-Polynomial of GCR as

$$M(\mathrm{GCR};x,y)=\sum_{i\leq j}\mu_{\left(i,j\right)}x^{i}y^{j}=\mu_{\left(4,6\right)}x^{4}y^{6}+\mu_{\left(4,9\right)}x^{4}y^{9}+\mu_{\left(4,13\right)}x^{4}y^{13}+\mu_{\left(4,18\right)}x^{4}y^{18}+\mu_{\left(6,9\right)}x^{6}y^{9}+\mu_{\left(9,9\right)}x^{9}y^{9}+\mu_{\left(9,13\right)}x^{9}y^{13}+\mu_{\left(13,13\right)}x^{13}y^{13}+\mu_{\left(13,18\right)}x^{13}y^{18}+\mu_{\left(18,18\right)}x^{18}y^{18}$$

This implies

(12) $$M(\mathrm{GCR};x,y)=24x^{4}y^{6}+[20(r+s+t)-120]x^{4}y^{9}+[16(rs+st+rt)-64(r+s+t)+192]x^{4}y^{13}+[12rst-24(rs+st+rt)+48(r+s+t)-96]x^{4}y^{18}+24x^{6}y^{9}+[4(r+s+t)-36]x^{9}y^{9}+[8(r+s+t)-48]x^{9}y^{13}+[4(rs+st+rt)-20(r+s+t)+72]x^{13}y^{13}+[2(rs+st+rt)-8(r+s+t)+24]x^{13}y^{18}+[3rst-7(rs+st+rt)+16(r+s+t)-36]x^{18}y^{18}$$

 □

Theorem 2 *If* GCR *is a graph of gold crystal, then the differential operators for* GCR(x,y) *are*

$$D_{x}(M(\mathrm{GCR};x,y))=96x^{4}y^{6}+[80(r+s+t)-480]x^{4}y^{9}+[64(rs+st+rt)-256(r+s+t)+768]x^{4}y^{13}+[48rst-96(rs+st+rt)+192(r+s+t)-384]x^{4}y^{18}+144x^{6}y^{9}+[36(r+s+t)-324]x^{9}y^{9}+[72(r+s+t)-432]x^{9}y^{13}+[52(rs+st+rt)-260(r+s+t)+936]x^{13}y^{13}+[26(rs+st+rt)-104(r+s+t)+312]x^{13}y^{18}+[54rst-126(rs+st+rt)+288(r+s+t)-648]x^{18}y^{18}$$

*and*

$$D_{y}(M(\mathrm{GCR};x,y))=144x^{4}y^{6}+[180(r+s+t)-1080]x^{4}y^{9}+[208(rs+st+rt)-832(r+s+t)+2496]x^{4}y^{13}+[216rst-432(rs+st+rt)+864(r+s+t)-1728]x^{4}y^{18}+216x^{6}y^{9}+[36(r+s+t)-324]x^{9}y^{9}+[104(r+s+t)-624]x^{9}y^{13}+[52(rs+st+rt)-260(r+s+t)+936]x^{13}y^{13}+[36(rs+st+rt)-144(r+s+t)+432]x^{13}y^{18}+[54rst-126(rs+st+rt)+288(r+s+t)-648]x^{18}y^{18}$$

Proof In view of Theorem 1 and using Equation (8), for the required outcome $D_{x}(M(\mathrm{GCR};x,y))$ for the structure of gold crystal.

$$D_{x}(M(\mathrm{GCR};x,y))=x\frac{\partial M(\mathrm{GCR};x,y))}{\partial x}=x\frac{\partial }{\partial x}(4x^{4}y^{6}+[20(r+s+t)-120]x^{4}y^{9}+[16(rs+st+rt)-64(r+s+t)+192]x^{4}y^{13}+[12rst-24(rs+st+rt)+48(r+s+t)-96]x^{4}y^{18}+24x^{6}y^{9}+[4(r+s+t)-36]x^{9}y^{9}+[8(r+s+t)-48]x^{9}y^{13}+[4(rs+st+rt)-20(r+s+t)+72]x^{13}y^{13}+[2(rs+st+rt)-8(r+s+t)+24]x^{13}y^{18}+[3rst-7(rs+st+rt)+16(r+s+t)-36]x^{18}y^{18})D_{x}(M(\mathrm{GCR};x,y))=x\frac{\partial }{\partial x}4x^{4}y^{6}+x\frac{\partial }{\partial x}[20(r+s+t)-120]x^{4}y^{9}+x\frac{\partial }{\partial x}[16(rs+st+rt)-64(r+s+t)+192]x^{4}y^{13}+x\frac{\partial }{\partial x}[12rst-24(rs+st+rt)+48(r+s+t)-96]x^{4}y^{18}+x\frac{\partial }{\partial x}24x^{6}y^{9}+x\frac{\partial }{\partial x}[4(r+s+t)-36]x^{9}y^{9}+x\frac{\partial }{\partial x}[8(r+s+t)-48]x^{9}y^{13}+x\frac{\partial }{\partial x}[4(rs+st+rt)-20(r+s+t)+72]x^{13}y^{13}+x\frac{\partial }{\partial x}[2(rs+st+rt)-8(r+s+t)+24]x^{13}y^{18}+x\frac{\partial }{\partial x}[3rst-7(rs+st+rt)+16(r+s+t)-36]x^{18}y^{18}$$

After applying differential operator formula (8), we have

(13) $$D_{x}(M(\mathrm{GCR};x,y))=96x^{4}y^{6}+[80(r+s+t)-480]x^{4}y^{9}+[64(rs+st+rt)-256(r+s+t)+768]x^{4}y^{13}+[48rst-96(rs+st+rt)+192(r+s+t)-384]x^{4}y^{18}+144x^{6}y^{9}+[36(r+s+t)-324]x^{9}y^{9}+[72(r+s+t)-432]x^{9}y^{13}+[52(rs+st+rt)-260(r+s+t)+936]x^{13}y^{13}+[26(rs+st+rt)-104(r+s+t)+312]x^{13}y^{18}+[54rst-126(rs+st+rt)+288(r+s+t)-648]x^{18}y^{18}$$

Similarly, using Equation (9) along with Equation (12) the required outcome $D_{y}(M(\mathrm{GCR};x,y))$ for GCR is:

$$D_{y}(M(\mathrm{GCR};x,y))=y\frac{\partial M(\mathrm{GCR};x,y))}{\partial y}=y\frac{\partial }{\partial y}(4x^{4}y^{6}+[20(r+s+t)-120]x^{4}y^{9}+[16(rs+st+rt)-64(r+s+t)+192]x^{4}y^{13}+[12rst-24(rs+st+rt)+48(r+s+t)-96]x^{4}y^{18}+24x^{6}y^{9}+[4(r+s+t)-36]x^{9}y^{9}+[8(r+s+t)-48]x^{9}y^{13}+[4(rs+st+rt)-20(r+s+t)+72]x^{13}y^{13}+[2(rs+st+rt)-8(r+s+t)+24]x^{13}y^{18}+[3rst-7(rs+st+rt)+16(r+s+t)-36]x^{18}y^{18}\;D_{y}(M(\mathrm{GCR};x,y))=y\frac{\partial }{\partial y}4x^{4}y^{6}+y\frac{\partial }{\partial y}[20(r+s+t)-120]x^{4}y^{9}+y\frac{\partial }{\partial y}[16(rs+st+rt)-64(r+s+t)+192]x^{4}y^{13}+y\frac{\partial }{\partial y}[12rst-24(rs+st+rt)+48(r+s+t)-96]x^{4}y^{18}+y\frac{\partial }{\partial y}24x^{6}y^{9}+y\frac{\partial }{\partial y}[4(r+s+t)-36]x^{9}y^{9}+y\frac{\partial }{\partial y}[8(r+s+t)-48]x^{9}y^{13}+y\frac{\partial }{\partial y}[4(rs+st+rt)-20(r+s+t)+72]x^{13}y^{13}+y\frac{\partial }{\partial y}[2(rs+st+rt)-8(r+s+t)+24]x^{13}y^{18}+y\frac{\partial }{\partial y}[3rst-7(rs+st+rt)+16(r+s+t)-36]x^{18}y^{18}$$

After applying differential operator formula (9), we have

(14) $$D_{y}(M(\mathrm{GCR};x,y))=144x^{4}y^{6}+[180(r+s+t)-1080]x^{4}y^{9}+[208(rs+st+rt)-832(r+s+t)+2496]x^{4}y^{13}+[216rst-432(rs+st+rt)+864(r+s+t)-1728]x^{4}y^{18}+216x^{6}y^{9}+[36(r+s+t)-324]x^{9}y^{9}+[104(r+s+t)-624]x^{9}y^{13}+[52(rs+st+rt)-260(r+s+t)+936]x^{13}y^{13}+[36(rs+st+rt)-144(r+s+t)+432]x^{13}y^{18}+[54rst-126(rs+st+rt)+)-648]x^{18}y^{18}$$

 □

Theorem 3 *If* GCR *be a graph of gold crystal, then the integral operators for* GCR(x,y) *are*

$$I_{x}(M(\mathrm{GCR};x,y)))=6x^{4}y^{6}+[5(r+s+t)-30]x^{4}y^{9}+[4(rs+st+rt)-16(r+s+t)+48]x^{4}y^{13}+[3rst-6(rs+st+rt)+12(r+s+t)-24]x^{4}y^{18}+4x^{6}y^{9}+[\frac{4}{9}(r+s+t)-4]x^{9}y^{9}+[\frac{8}{9}(r+s+t)-\frac{48}{9}]x^{9}y^{13}+[\frac{4}{13}(rs+st+rt)-\frac{20}{13}(r+s+t)+\frac{72}{13}]x^{13}y^{13}+[\frac{2}{13}(rs+st+rt)-\frac{8}{13}(r+s+t)+\frac{24}{13}]x^{13}y^{18}+[\frac{1}{6}rst-\frac{7}{18}(rs+st+rt)+\frac{8}{9}(r+s+t)-2]x^{18}y^{18}$$

*and*

$$I_{y}(M(\mathrm{GCR};x,y)))=4x^{4}y^{6}+[\frac{20}{9}(r+s+t)-\frac{120}{9}]x^{4}y^{9}+[\frac{16}{13}(rs+st+rt)-\frac{64}{13}(r+s+t)+\frac{192}{13}]x^{4}y^{13}+[\frac{2}{3}rst-\frac{4}{3}(rs+st+rt)+\frac{8}{3}(r+s+t)-\frac{16}{3}]x^{4}y^{18}+\frac{24}{9}x^{6}y^{9}+[\frac{4}{9}(r+s+t)-4]x^{9}y^{9}+[\frac{8}{13}(r+s+t)-\frac{48}{13}]x^{9}y^{13}+[\frac{4}{13}(rs+st+rt)-\frac{20}{13}(r+s+t)+\frac{72}{13}]x^{13}y^{13}+[\frac{1}{9}(rs+st+rt)-\frac{4}{9}(r+s+t)+\frac{4}{3}]x^{13}y^{18}+[\frac{1}{6}rst-\frac{7}{18}(rs+st+rt)+\frac{8}{9}(r+s+t)-2]x^{18}y^{18}$$

Proof In view of Theorem 1 and using Equation (10), for the required outcome $I_{x}(M(\mathrm{GCR};x,y))$ for the structure of gold crystal.

$$I_{x}(M(\mathrm{GCR};x,y)))=\int_{0}^{x}\frac{M(\mathrm{GCR};z,y))}{z}dz$$

$$I_{x}(M(\mathrm{GCR};x,y)))=\int_{0}^{x}\frac{1}{z}[24z^{4}y^{6}+[20(r+s+t)-120]z^{4}y^{9}+[16(rs+st+rt)-64(r+s+t)+192]z^{4}y^{13}+[12rst-24(rs+st+rt)+48(r+s+t)-96]z^{4}y^{18}+24z^{6}y^{9}+[4(r+s+t)-36]z^{9}y^{9}+[8(r+s+t)-48]z^{9}y^{13}+[4(rs+st+rt)-20(r+s+t)+72]z^{13}y^{13}+[2(rs+st+rt)-8(r+s+t)+24]z^{13}y^{18}+[3rst-7(rs+st+rt)+16(r+s+t)-36]z^{18}y^{18}]dz$$

Implementing Integral operator formula (10), we obtain

$$I_{x}(M(\mathrm{GCR};x,y)))=\int_{0}^{x}24z^{3}y^{6}dz+\int_{0}^{x}[20(r+s+t)-120]z^{3}y^{9}dz+\int_{0}^{x}[16(rs+st+rt)-64(r+s+t)+192]z^{3}y^{13}dz+\int_{0}^{x}[12rst-24(rs+st+rt)+48(r+s+t)-96]z^{3}y^{18}dz+\int_{0}^{x}24z^{5}y^{9}dz+\int_{0}^{x}[4(r+s+t)-36]z^{8}y^{9}dz+\int_{0}^{x}[8(r+s+t)-48]z^{8}y^{13}dz+\int_{0}^{x}[4(rs+st+rt)-20(r+s+t)+72]z^{12}y^{13}dz+\int_{0}^{x}[2(rs+st+rt)-8(r+s+t)+24]z^{12}y^{18}dz+\int_{0}^{x}[3rst-7(rs+st+rt)+16(r+s+t)-36]z^{17}y^{18}dz$$

$$I_{x}(M(\mathrm{GCR};x,y)))=\frac{1}{4}24z^{4}y^{6}{|}_{0}^{x}+\frac{1}{4}[20(r+s+t)-120]z^{4}y^{9}{|}_{0}^{x}+\frac{1}{4}[16(rs+st+rt)-64(r+s+t)+192]z^{4}y^{13}{|}_{0}^{x}+\frac{1}{4}[12rst-24(rs+st+rt)+48(r+s+t)-96]z^{4}y^{18}{|}_{0}^{x}+\frac{1}{6}24z^{6}y^{9}{|}_{0}^{x}+\frac{1}{9}[4(r+s+t)-36]z^{9}y^{9}+\frac{1}{9}[8(r+s+t)-48]z^{9}y^{13}{|}_{0}^{x}+\frac{1}{13}[4(rs+st+rt)-20(r+s+t)+72]z^{13}y^{13}{|}_{0}^{x}+\frac{1}{13}[2(rs+st+rt)-8(r+s+t)+24]z^{13}y^{18}{|}_{0}^{x}+\frac{1}{18}[3rst-7(rs+st+rt)+16(r+s+t)-36]z^{18}y^{18}{|}_{0}^{x}$$

After simplification, we get

$$I_{x}(M(\mathrm{GCR};x,y)))=6x^{4}y^{6}+[5(r+s+t)-30]x^{4}y^{9}+[4(rs+st+rt)-16(r+s+t)+48]x^{4}y^{13}+[3rst-6(rs+st+rt)+12(r+s+t)-24]x^{4}y^{18}+4x^{6}y^{9}+[\frac{4}{9}(r+s+t)-4]x^{9}y^{9}+[\frac{8}{9}(r+s+t)-\frac{48}{9}]x^{9}y^{13}+[\frac{4}{13}(rs+st+rt)-\frac{20}{13}(r+s+t)+\frac{72}{13}]x^{13}y^{13}+[\frac{2}{13}(rs+st+rt)-\frac{8}{13}(r+s+t)+\frac{24}{13}]x^{13}y^{18}+[\frac{1}{6}rst-\frac{7}{18}(rs+st+rt)+\frac{8}{9}(r+s+t)-2]x^{18}y^{18}$$

Similarly, using Equation (11) along with Equation (12) for the required outcome $I_{y}(M(\mathrm{GCR};x,y))$ for the structure of gold crystal GCR.

$$I_{y}(M(\mathrm{GCR};x,y))))=\int_{0}^{y}\frac{M(\mathrm{GCR};x,z))))}{z}dz\;I_{y}(M(\mathrm{GCR};x,y))))=\int_{0}^{y}\frac{1}{z}(24x^{4}z^{6}+[20(r+s+t)-120]x^{4}z^{9}+[16(rs+st+rt)-64(r+s+t)+192]x^{4}z^{13}+[12rst-24(rs+st+rt)+48(r+s+t)-96]x^{4}z^{18}+24x^{6}y^{9}+[4(r+s+t)-36]x^{9}z^{9}+[8(r+s+t)-48]x^{9}z^{13}+[4(rs+st+rt)-20(r+s+t)+72]x^{13}z^{13}+[2(rs+st+rt)-8(r+s+t)+24]x^{13}z^{18}+[3rst-7(rs+st+rt)+16(r+s+t)-36]x^{18}z^{18})dz$$

Implementing Integral on each component

$$I_{y}(M(\mathrm{GCR};x,y))))=\int_{0}^{y}24x^{4}z^{5}dz+\int_{0}^{y}[20(r+s+t)-120]x^{4}z^{8}dz+\int_{0}^{y}[16(rs+st+rt)-64(r+s+t)+192]x^{4}z^{12}dz+\int_{0}^{y}[12rst-24(rs+st+rt)+48(r+s+t)-96]x^{4}z^{17}dz+\int_{0}^{y}24x^{6}y^{8}dz+\int_{0}^{y}[4(r+s+t)-36]x^{9}z^{8}dz+\int_{0}^{y}[8(r+s+t)-48]x^{9}z^{12}dz+\int_{0}^{y}[4(rs+st+rt)-20(r+s+t)+72]x^{13}z^{12}dz+\int_{0}^{y}[2(rs+st+rt)-8(r+s+t)+24]x^{13}z^{17}dz+\int_{0}^{y}[3rst-7(rs+st+rt)+16(r+s+t)-36]x^{18}z^{17}dz$$

$$I_{y}(M(\mathrm{GCR};x,y))))=\frac{1}{6}24x^{4}z^{6}{|}_{0}^{y}+\frac{1}{9}[20(r+s+t)-120]x^{4}z^{9}{|}_{0}^{y}+\frac{1}{13}[16(rs+st+rt)-64(r+s+t)+192]x^{4}z^{13}{|}_{0}^{y}+\frac{1}{18}[12rst-24(rs+st+rt)+48(r+s+t)-96]x^{4}z^{18}{|}_{0}^{y}+\frac{1}{9}24x^{6}z^{9}{|}_{0}^{y}+\frac{1}{9}[4(r+s+t)-36]x^{9}z^{9}{|}_{0}^{y}+\frac{1}{13}[8(r+s+t)-48]x^{9}z^{13}{|}_{0}^{y}+\frac{1}{13}[4(rs+st+rt)-20(r+s+t)+72]x^{13}z^{13}{|}_{0}^{y}+\frac{1}{18}[2(rs+st+rt)-8(r+s+t)+24]x^{13}z^{18}{|}_{0}^{y}+\frac{1}{18}[3rst-7(rs+st+rt)+16(r+s+t)-36]x^{18}z^{18}{|}_{0}^{y}$$

After simplification, we get

(15) $$I_{y}(M(\mathrm{GCR};x,y)))=4x^{4}y^{6}+[\frac{20}{9}(r+s+t)-\frac{120}{9}]x^{4}y^{9}+[\frac{16}{13}(rs+st+rt)-\frac{64}{13}(r+s+t)+\frac{192}{13}]x^{4}y^{13}+[\frac{2}{3}rst-\frac{4}{3}(rs+st+rt)+\frac{8}{3}(r+s+t)-\frac{16}{3}]x^{4}y^{18}+\frac{24}{9}x^{6}y^{9}+[\frac{4}{9}(r+s+t)-4]x^{9}y^{9}+[\frac{8}{13}(r+s+t)-\frac{48}{13}]x^{9}y^{13}+[\frac{4}{13}(rs+st+rt)-\frac{20}{13}(r+s+t)+\frac{72}{13}]x^{13}y^{13}+[\frac{1}{9}(rs+st+rt)-\frac{4}{9}(r+s+t)+\frac{4}{3}]x^{13}y^{18}+[\frac{1}{6}rst-\frac{7}{18}(rs+st+rt)+\frac{8}{9}(r+s+t)-2]x^{18}y^{18}$$

 □

Theorem 4 *If* GCR *be graph of gold crystal, then the First Zagreb* M *-Polynomial for* GCR *is*

$$M_{M_{1}}(\mathrm{GCR};x,y))=240x^{4}y^{6}+[260(r+s+t)-1560]x^{4}y^{9}+[272(rs+st+rt)-1088(r+s+t)+3264]x^{4}y^{13}+[264rst-528(rs+st+rt)+1056(r+s+t)-2112]x^{4}y^{18}+360x^{6}y^{9}+[72(r+s+t)-648]x^{9}y^{9}+[176(r+s+t)-1056]x^{9}y^{13}+[104(rs+st+rt)-520(r+s+t)+1872]x^{13}y^{13}+[62(rs+st+rt)-248(r+s+t)+744]x^{13}y^{18}+[108rst-252(rs+st+rt)+576(r+s+t)-1296]x^{18}y^{18}$$

Proof The First Zagreb M-Polynomial is determined by using Equation (4), along with Equation (2). We get the required assertion by using Equation (13) and Equation (14), which reveals the differential operator function for the GCR.

The article "Computation of differential and integral operators using ℳ-polynomials of gold crystal" was retracted in 2025. Reasons: plagiarism; unreliable results or conclusions; concerns about the peer review; concerns about the citations.

Now using Equation (4), we have

$$M_{M_{1}}(\mathrm{GCR};x,y))=(D_{x}+D_{y})(M(\mathrm{GCR};x,y))=D_{x}(M(\mathrm{GCR};x,y))+D_{y}(M(\mathrm{GCR};x,y))=96x^{4}y^{6}+[80(r+s+t)-480]x^{4}y^{9}+[64(rs+st+rt)-256(r+s+t)+768]x^{4}y^{13}+[48rst-96(rs+st+rt)+192(r+s+t)-384]x^{4}y^{18}+144x^{6}y^{9}+[36(r+s+t)-324]x^{9}y^{9}+[72(r+s+t)-432]x^{9}y^{13}+[52(rs+st+rt)-260(r+s+t)+936]x^{13}y^{13}+[26(rs+st+rt)-104(r+s+t)+312]x^{13}y^{18}+[54rst-126(rs+st+rt)+288(r+s+t)-648]x^{18}y^{18}+144x^{4}y^{6}+[180(r+s+t)-1080]x^{4}y^{9}+[208(rs+st+rt)-832(r+s+t)+2496]x^{4}y^{13}+[216rst-432(rs+st+rt)+864(r+s+t)-1728]x^{4}y^{18}+216x^{6}y^{9}+[36(r+s+t)-324]x^{9}y^{9}+[104(r+s+t)-624]x^{9}y^{13}+[52(rs+st+rt)-260(r+s+t)+936]x^{13}y^{13}+[36(rs+st+rt)-144(r+s+t)+432]x^{13}y^{18}+[54rst-126(rs+st+rt)+288(r+s+t)-648]x^{18}y^{18}$$

This gives

$$M_{M_{1}}(\mathrm{GCR};x,y))=240x^{4}y^{6}+[260(r+s+t)-1560]x^{4}y^{9}+[272(rs+st+rt)-1088(r+s+t)+3264]x^{4}y^{13}+[264rst-528(rs+st+rt)+1056(r+s+t)-2112]x^{4}y^{18}+360x^{6}y^{9}+[72(r+s+t)-648]x^{9}y^{9}+[176(r+s+t)-1056]x^{9}y^{13}+[104(rs+st+rt)-520(r+s+t)+1872]x^{13}y^{13}+[62(rs+st+rt)-248(r+s+t)+744]x^{13}y^{18}+[108rst-252(rs+st+rt)+576(r+s+t)-1296]x^{18}y^{18}$$

 □

Theorem 5 *If* GCR *is a graph of gold crystal, then the Second Zagreb* M *-Polynomial for* GCR *is*

$$M_{M_{2}}((\mathrm{GCR};x,y))=15xy^{3}+8xy^{4}+16x^{2}y^{2}+66x^{2}y^{3}+8x^{2}y^{4}+18x^{3}y^{3}+12x^{3}y^{4}$$

Proof The Second Zagreb M-Polynomial is determined using Equation (5) and Equation (3). We get the required assertion using Equation (13) and Equation (14), which reveals the differential operator function for GCR. Using formula in Equation (5), we get

$$M_{M_{2}}(\mathrm{GCR})=(D_{x}.D_{y})(M(\mathrm{GCR};x,y))=D_{x}[(D_{y})(M(\mathrm{GCR};x,y))]$$

From the Equation (14), we have

$$M_{M_{2}}(\mathrm{GCR})=D_{x}(144x^{4}y^{6}+[180(r+s+t)-1080]x^{4}y^{9}+[208(rs+st+rt)-832(r+s+t)+2496]x^{4}y^{13}+[216rst-432(rs+st+rt)+864(r+s+t)-1728]x^{4}y^{18}+216x^{6}y^{9}+[36(r+s+t)-324]x^{9}y^{9}+[104(r+s+t)-624]x^{9}y^{13}+[52(rs+st+rt)-260(r+s+t)+936]x^{13}y^{13}+[36(rs+st+rt)-144(r+s+t)+432]x^{13}y^{18}+[54rst-126(rs+st+rt)+288(r+s+t)-648]x^{18}y^{18})M_{M_{2}}(\mathrm{GCR})=x\frac{\partial }{\partial x}144x^{4}y^{6}+x\frac{\partial }{\partial x}[180(r+s+t)-1080]x^{4}y^{9}+x\frac{\partial }{\partial x}[208(rs+st+rt)-832(r+s+t)+2496]x^{4}y^{13}+x\frac{\partial }{\partial x}[216rst-432(rs+st+rt)+864(r+s+t)-1728]x^{4}y^{18}+x\frac{\partial }{\partial x}216x^{6}y^{9}+x\frac{\partial }{\partial x}[36(r+s+t)-324]x^{9}y^{9}+[104(r+s+t)-624]x^{9}y^{13}+x\frac{\partial }{\partial x}[52(rs+st+rt)-260(r+s+t)+936]x^{13}y^{13}+x\frac{\partial }{\partial x}[36(rs+st+rt)-144(r+s+t)+432]x^{13}y^{18}+x\frac{\partial }{\partial x}[54rst-126(rs+st+rt)+288(r+s+t)-648]x^{18}y^{18}$$

After taking partial derivatives, we get

$$M_{M_{2}}(\mathrm{GCR};x,y))=576x^{4}y^{6}+[720(r+s+t)-4320]x^{4}y^{9}+[832(rs+st+rt)-3328(r+s+t)+9984]x^{4}y^{13}+[864rst-1728(rs+st+rt)+3456(r+s+t)-6912]x^{4}y^{18}+1296x^{6}y^{9}+[324(r+s+t)-2916]x^{9}y^{9}+[936(r+s+t)-5616]x^{9}y^{13}+[676(rs+st+rt)-3380(r+s+t)+12168]x^{13}y^{13}+[468(rs+st+rt)-1872(r+s+t)+5616]x^{13}y^{18}+[972rst-2268(rs+st+rt)+5184(r+s+t)-11664]x^{18}y^{18}$$

 □

Theorem 6 *If* GCR *is a graph of gold crystal, then the General Randic* M *-Polynomial for* GCR(x,y) *is*

$$M_{R_{\alpha }}((\mathrm{GCR};x,y))={\left(24\right)}^{\alpha }.24x^{4}y^{6}+{\left(36\right)}^{\alpha }[20(r+s+t)-120]x^{4}y^{9}+{\left(52\right)}^{\alpha }[16(rs+st+rt)-64(r+s+t)+192]x^{4}y^{13}+{\left(72\right)}^{\alpha }[12rst-24(rs+st+rt)+48(r+s+t)-96]x^{4}y^{18}+{\left(54\right)}^{\alpha }24x^{6}y^{9}+{\left(81\right)}^{\alpha }[4(r+s+t)-36]x^{9}y^{9}+{\left(117\right)}^{\alpha }[8(r+s+t)-48]x^{9}y^{13}+{\left(169\right)}^{\alpha }[4(rs+st+rt)-20(r+s+t)+72]x^{13}y^{13}+{\left(234\right)}^{\alpha }[2(rs+st+rt)-8(r+s+t)+24]x^{13}y^{18}+{\left(324\right)}^{\alpha }[3rst-7(rs+st+rt)+16(r+s+t)-36]x^{18}y^{18}$$

Proof The General Randic M-Polynomial is obtained by using Equation (6) and Equation (7) along with Equation (13) and Equation (14)

$$M_{R_{\alpha }}(\mathrm{GCR})=(D_{x}^{\alpha }D_{y}^{\alpha })(M(\mathrm{GCR};x,y))M_{R_{\alpha }}(\mathrm{GCR})=D_{x}^{\alpha }D_{y}^{\alpha }(24x^{4}y^{6}+[20(r+s+t)-120]x^{4}y^{9}+[16(rs+st+rt)-64(r+s+t)+192]x^{4}y^{13}+[12rst-24(rs+st+rt)+48(r+s+t)-96]x^{4}y^{18}+24x^{6}y^{9}+[4(r+s+t)-36]x^{9}y^{9}+[8(r+s+t)-48]x^{9}y^{13}+[4(rs+st+rt)-20(r+s+t)+72]x^{13}y^{13}+[2(rs+st+rt)-8(r+s+t)+24]x^{13}y^{18}+[3rst-7(rs+st+rt)+16(r+s+t)-36]x^{18}y^{18})M_{R_{\alpha }}(\mathrm{GCR})=(D_{x}^{\alpha })({\left(6\right)}^{\alpha }24x^{4}y^{6}+{\left(9\right)}^{\alpha }[20(r+s+t)-120]x^{4}y^{9}+{\left(13\right)}^{\alpha }[16(rs+st+rt)-64(r+s+t)+192]x^{4}y^{13}+{\left(18\right)}^{\alpha }[12rst-24(rs+st+rt)+48(r+s+t)-96]x^{4}y^{18}+{\left(9\right)}^{\alpha }24x^{6}y^{9}+{\left(9\right)}^{\alpha }[4(r+s+t)-36]x^{9}y^{9}+{\left(13\right)}^{\alpha }[8(r+s+t)-48]x^{9}y^{13}+{\left(13\right)}^{\alpha }[4(rs+st+rt)-20(r+s+t)+72]x^{13}y^{13}+{\left(18\right)}^{\alpha }[2(rs+st+rt)-8(r+s+t)+24]x^{13}y^{18}+{\left(18\right)}^{\alpha }[3rst-7(rs+st+rt)+16(r+s+t)-36]x^{18}y^{18}$$

$$M_{R_{\alpha }}((\mathrm{GCR};x,y))={\left(24\right)}^{\alpha }.24x^{4}y^{6}+{\left(36\right)}^{\alpha }[20(r+s+t)-120]x^{4}y^{9}+{\left(52\right)}^{\alpha }[16(rs+st+rt)-64(r+s+t)+192]x^{4}y^{13}+{\left(72\right)}^{\alpha }[12rst-24(rs+st+rt)+48(r+s+t)-96]x^{4}y^{18}+{\left(54\right)}^{\alpha }24x^{6}y^{9}+{\left(81\right)}^{\alpha }[4(r+s+t)-36]x^{9}y^{9}+{\left(117\right)}^{\alpha }[8(r+s+t)-48]x^{9}y^{13}+{\left(169\right)}^{\alpha }[4(rs+st+rt)-20(r+s+t)+72]x^{13}y^{13}+{\left(234\right)}^{\alpha }[2(rs+st+rt)-8(r+s+t)+24]x^{13}y^{18}+{\left(324\right)}^{\alpha }[3rst-7(rs+st+rt)+16(r+s+t)-36]x^{18}y^{18}$$

 □

The article "Computation of differential and integral operators using ℳ-polynomials of gold crystal" was retracted in 2025. Reasons: plagiarism; unreliable results or conclusions; concerns about the peer review; concerns about the citations.

## 3 Topological indices for Gold Crystal

In this section, we compute topological indices of GCR by using the corresponding M-Polynomial in Theorem 1. In the Table 2

$$D_{x}(f(x,y))=x\frac{\partial (f(x,y))}{\partial x}\;D_{y}(f(x,y))=y\frac{\partial (f(x,y))}{\partial y}\;I_{x}(f(x,y))=\int_{0}^{x}\frac{1}{z}(f(z,y))dz\;I_{y}(f(x,y))=\int_{0}^{y}\frac{1}{z}(f(x,z))dz\;J(f(x,y))=f(x,x)$$

Theorem 7 *If*GCR(x,y)*graph of gold crystal, then the First Zagreb Index of*GCR*is*

$$M_{1}(\mathrm{GCR})=372rst-342(rs+st+rt)+284(r+s+t)-192$$

**Table 2:** Formulation of TI's using M-Polynomial.

Topological index	Derivation From M(GCR)
*M*_1_	$(D_{x}+D_{y})(M(\mathrm{GCR})){|}_{x=y=1}$
*M*_2_	$(D_{x}D_{y})(M(\mathrm{GCR})){|}_{x=y=1}$
*HM*	${\left(D_{x}+D_{y}\right)}^{2}(M(\mathrm{GCR})){|}_{x=y=1}$
*σ*	${\left(D_{x}-D_{y}\right)}^{2}(M(\mathrm{GCR})){|}_{x=y=1}$
M2m	$(I_{x}I_{y})(M(\mathrm{GCR})){|}_{x=y=1}$
*R*_*α*_	$(D_{x}^{\alpha }D_{y}^{\alpha })(M(\mathrm{GCR})){|}_{x=y=1}$
*RR*_*α*_	$(I_{x}^{\alpha }I_{y}^{\alpha })(M(\mathrm{GCR})){|}_{x=y=1}$
*ReZG*_3_	$(D_{x}D_{y})(D_{x}+D_{y})(M(\mathrm{GCR})){|}_{x=y=1}$
*SDD*	$(D_{x}I_{y}+I_{x}D_{y})(M(\mathrm{GCR})){|}_{x=y=1}$
*H*	$2I_{x}J(M(\mathrm{GCR})){|}_{x=y=1}$
*I*	$I_{x}JD_{x}D_{y}(M(\mathrm{GCR})){|}_{x=y=1}$

Proof By adding Equation (13) and Equation (14), we get

$$D_{x}(M(\mathrm{GCR};x,y))+D_{y}(M(\mathrm{GCR};x,y))=96x^{4}y^{6}+[80(r+s+t)-480]x^{4}y^{9}+[64(rs+st+rt)-256(r+s+t)+768]x^{4}y^{13}+[48rst-96(rs+st+rt)+192(r+s+t)-384]x^{4}y^{18}+144x^{6}y^{9}+[36(r+s+t)-324]x^{9}y^{9}+[72(r+s+t)-432]x^{9}y^{13}+[52(rs+st+rt)-260(r+s+t)+936]x^{13}y^{13}+[26(rs+st+rt)-104(r+s+t)+312]x^{13}y^{18}+[54rst-126(rs+st+rt)+288(r+s+t)-648]x^{18}y^{18}+144x^{4}y^{6}+[180(r+s+t)-1080]x^{4}y^{9}+[208(rs+st+rt)-832(r+s+t)+2496]x^{4}y^{13}+[216rst-432(rs+st+rt)+864(r+s+t)-1728]x^{4}y^{18}+216x^{6}y^{9}+[36(r+s+t)-324]x^{9}y^{9}+[104(r+s+t)-624]x^{9}y^{13}+[52(rs+st+rt)-260(r+s+t)+936]x^{13}y^{13}+[36(rs+st+rt)-144(r+s+t)+432]x^{13}y^{18}+[54rst-126(rs+st+rt)+288(r+s+t)-648]x^{18}y^{18}(D_{x}+D_{y})(M(\mathrm{GCR};x,y))=240x^{4}y^{6}+[260(r+s+t)-1560]x^{4}y^{9}+[272(rs+st+rt)-1088(r+s+t)+3264]x^{4}y^{13}+[264rst-528(rs+st+rt)+1056(r+s+t)-2112]x^{4}y^{18}+360x^{6}y^{9}+[72(r+s+t)-648]x^{9}y^{9}+[176(r+s+t)-1056]x^{9}y^{13}+[104(rs+st+rt)-520(r+s+t)+1872]x^{13}y^{13}+[62(rs+st+rt)-248(r+s+t)+744]x^{13}y^{18}+[108rst-252(rs+st+rt)+576(r+s+t)-1296]x^{18}y^{18}(D_{x}+D_{y})(M(\mathrm{GCR};x,y)){|}_{x=y=1}=(240x^{4}y^{6}+[260(r+s+t)-1560]x^{4}y^{9}+[272(rs+st+rt)-1088(r+s+t)+3264]x^{4}y^{13}+[264rst-528(rs+st+rt)+1056(r+s+t)-2112]x^{4}y^{18}+360x^{6}y^{9}+[72(r+s+t)-648]x^{9}y^{9}+[176(r+s+t)-1056]x^{9}y^{13}+[104(rs+st+rt)-520(r+s+t)+1872]x^{13}y^{13}+[62(rs+st+rt)-248(r+s+t)+744]x^{13}y^{18}+[108rst-252(rs+st+rt)+576(r+s+t)-1296]x^{18}y^{18}){|}_{x=y=1}\;M_{1}(\mathrm{GCR}(x,y))=372rst-342(rs+st+rt)+284(r+s+t)-192$$

 □

Theorem 8 *If* GCR *is a graph of gold crystal, then the Second Zagreb Index for* GCR(x,y) *is*

$$M_{2}(\mathrm{GCR})=1836rst-2020(rs+st+rt)+2040(r+s+t)-1788$$

Proof In view of Table 2 along with equation (12) and Theorem 5, we get

$$M(\mathrm{GCR};x,y)=24x^{4}y^{6}+[20(r+s+t)-120]x^{4}y^{9}+[16(rs+st+rt)-64(r+s+t)+192]x^{4}y^{13}+[12rst-24(rs+st+rt)+48(r+s+t)-96]x^{4}y^{18}+24x^{6}y^{9}+[4(r+s+t)-36]x^{9}y^{9}+[8(r+s+t)-48]x^{9}y^{13}+[4(rs+st+rt)-20(r+s+t)+72]x^{13}y^{13}+[2(rs+st+rt)-8(r+s+t)+24]x^{13}y^{18}+[3rst-7(rs+st+rt)+16(r+s+t)-36]x^{18}y^{18}\;D_{x}[(D_{y}(M(\mathrm{GCR};x,y))]=D_{x}(144x^{4}y^{6}+[180(r+s+t)-1080]x^{4}y^{9}+[208(rs+st+rt)-832(r+s+t)+2496]x^{4}y^{13}+[216rst-432(rs+st+rt)+864(r+s+t)-1728]x^{4}y^{18}+216x^{6}y^{9}+[36(r+s+t)-324]x^{9}y^{9}+[104(r+s+t)-624]x^{9}y^{13}+[52(rs+st+rt)-260(r+s+t)+936]x^{13}y^{13}+[36(rs+st+rt)-144(r+s+t)+432]x^{13}y^{18}+[54rst-126(rs+st+rt)+288(r+s+t)-648]x^{18}y^{18})(D_{x}D_{y})(M(\mathrm{GCR};x,y))=576x^{4}y^{6}+[720(r+s+t)-4320]x^{4}y^{9}+[832(rs+st+rt)-3328(r+s+t)+9984]x^{4}y^{13}+[864rst-1728(rs+st+rt)+3456(r+s+t)-6912]x^{4}y^{18}+1296x^{6}y^{9}+[324(r+s+t)-2916]x^{9}y^{9}+[936(r+s+t)-5616]x^{9}y^{13}+[676(rs+st+rt)-3380(r+s+t)+12168]x^{13}y^{13}+[468(rs+st+rt)-1872(r+s+t)+5616]x^{13}y^{18}+[972rst-2268(rs+st+rt)+5184(r+s+t)-11664]x^{18}y^{18}(D_{x}D_{y})(M(\mathrm{GCR};x,y)){|}_{x=y=1}=(576x^{4}y^{6}+[720(r+s+t)-4320]x^{4}y^{9}+[832(rs+st+rt)-3328(r+s+t)+9984]x^{4}y^{13}+[864rst-1728(rs+st+rt)+3456(r+s+t)-6912]x^{4}y^{18}+1296x^{6}y^{9}+[324(r+s+t)-2916]x^{9}y^{9}+[936(r+s+t)-5616]x^{9}y^{13}+[676(rs+st+rt)-3380(r+s+t)+12168]x^{13}y^{13}+[468(rs+st+rt)-1872(r+s+t)+5616]x^{13}y^{18}+[972rst-2268(rs+st+rt)+5184(r+s+t)-11664]x^{18}y^{18}){|}_{x=y=1}\;M_{2}(\mathrm{GCR})=1836rst-2020(rs+st+rt)+2040(r+s+t)-1788$$

 □

Theorem 9 *If* GCR *is a graph of gold crystal, then the Hyper Zagreb Index of* GCR(x,y) *is*

HM(GCR)=9696rst−11438(rs+st+rt)+12812(r+s+t)−13272

Proof In the view of Table 2, we have

$$D_{x}^{2}(M(\mathrm{GCR};x,y))=384x^{4}y^{6}+[320(r+s+t)-1920]x^{4}y^{9}+[256(rs+st+rt)-1024(r+s+t)+3072]x^{4}y^{13}+864x^{6}y^{9}+[192rst-384(rs+st+rt)+768(r+s+t)-1536]x^{4}y^{18}+[324(r+s+t)-2916]x^{9}y^{9}+[648(r+s+t)-3888]x^{9}y^{13}+[676(rs+st+rt)-3380(r+s+t)+12168]x^{13}y^{13}+[338(rs+st+rt)-1352(r+s+t)+4056]x^{13}y^{18}+[972rst-2268(rs+st+rt)+5184(r+s+t)-11664]x^{18}y^{18}\;D_{y}^{2}(M(\mathrm{GCR};x,y))=864x^{4}y^{6}+[1620(r+s+t)-9720]x^{4}y^{9}+[2704(rs+st+rt)-10816(r+s+t)+32448]x^{4}y^{13}+1944x^{6}y^{9}+[3888rst-7776(rs+st+rt)+15552(r+s+t)-31104]x^{4}y^{18}+[324(r+s+t)-2916]x^{9}y^{9}+[1352(r+s+t)-8112]x^{9}y^{13}+[676(rs+st+rt)-3380(r+s+t)+12168]x^{13}y^{13}+[648(rs+st+rt)-2592(r+s+t)+7776]x^{13}y^{18}+[972rst-2268(rs+st+rt)+5184(r+s+t)-11664]x^{18}y^{18}(2D_{x}D_{y})(M(\mathrm{GCR};x,y))=1152x^{4}y^{6}+[1440(r+s+t)-8640]x^{4}y^{9}+[1664(rs+st+rt)-6656(r+s+t)+19968]x^{4}y^{13}+2592x^{6}y^{9}+[1728rst-3456(rs+st+rt)+6912(r+s+t)-13824]x^{4}y^{18}+[648(r+s+t)-5832]x^{9}y^{9}+[1872(r+s+t)-11232]x^{9}y^{13}+[1352(rs+st+rt)-6760(r+s+t)+24336]x^{13}y^{13}+[936(rs+st+rt)-3744(r+s+t)+11232]x^{13}y^{18}+[1944rst-4536(rs+st+rt)+10368(r+s+t)-23328]x^{18}y^{18}(D_{x}^{2}+D_{y}^{2}+2D_{x}D_{y})(M(\mathrm{GCR};x,y)){|}_{x=y=1}=(2400x^{4}y^{6}+[3380(r+s+t)-20280]x^{4}y^{9}+[4624(rs+st+rt)-18496(r+s+t)+55488]x^{4}y^{13}+5400x^{6}y^{9}+[5808rst-11616(rs+st+rt)+23232(r+s+t)-46464]x^{4}y^{18}+[1296(r+s+t)-11664]x^{9}y^{9}+[3872(r+s+t)-23232]x^{9}y^{13}+[2704(rs+st+rt)-13520(r+s+t)+48672]x^{13}y^{13}+[1922(rs+st+rt)-7688(r+s+t)+23064]x^{13}y^{18}+[3888rst-9072(rs+st+rt)+20736(r+s+t)-46656]x^{18}y^{18}){|}_{x=y=1}$$

After putting limits, we have

HM(GCR)=9696rst−11438(rs+st+rt)+12812(r+s+t)−13272

 □

Theorem 10 *If* GCR *is a graph of gold crystal, then the Sigma Index for* M *-Polynomial of* GCR(x,y) *is*

σ(GCR)=2352rst−3358(rs+st+rt)+4652(r+s+t)−6120

Proof In the view Table 2 and after apply differential operator on Equation (13) and Equation (14), we have

$$D_{x}^{2}(M(\mathrm{GCR};x,y))=384x^{4}y^{6}+[320(r+s+t)-1920]x^{4}y^{9}+[256(rs+st+rt)-1024(r+s+t)+3072]x^{4}y^{13}+[192rst-384(rs+st+rt)+768(r+s+t)-1536]x^{4}y^{18}+864x^{6}y^{9}+[324(r+s+t)-2916]x^{9}y^{9}+[648(r+s+t)-3888]x^{9}y^{13}+[676(rs+st+rt)-3380(r+s+t)+12168]x^{13}y^{13}+[338(rs+st+rt)-1352(r+s+t)+4056]x^{13}y^{18}+[972rst-2268(rs+st+rt)+5184(r+s+t)-11664]x^{18}y^{18}\;D_{y}^{2}(M(\mathrm{GCR};x,y))=864x^{4}y^{6}+[1620(r+s+t)-9720]x^{4}y^{9}+[2704(rs+st+rt)-10816(r+s+t)+32448]x^{4}y^{13}+[3888rst-7776(rs+st+rt)+15552(r+s+t)-31104]x^{4}y^{18}+1944x^{6}y^{9}+[324(r+s+t)-2916]x^{9}y^{9}+[1352(r+s+t)-8112]x^{9}y^{13}+[676(rs+st+rt)-3380(r+s+t)+12168]x^{13}y^{13}+[648(rs+st+rt)-2592(r+s+t)+7776]x^{13}y^{18}+[972rst-2268(rs+st+rt)+5184(r+s+t)-11664]x^{18}y^{18}(2D_{x}D_{y})(M(\mathrm{GCR};x,y))=1152x^{4}y^{6}+[1440(r+s+t)-8640]x^{4}y^{9}+[1664(rs+st+rt)-6656(r+s+t)+19968]x^{4}y^{13}+[1728rst-3456(rs+st+rt)+6912(r+s+t)-13824]x^{4}y^{18}+2592x^{6}y^{9}+[648(r+s+t)-5832]x^{9}y^{9}+[1872(r+s+t)-11232]x^{9}y^{13}+[1352(rs+st+rt)-6760(r+s+t)+24336]x^{13}y^{13}+[936(rs+st+rt)-3744(r+s+t)+11232]x^{13}y^{18}+[1944rst-4536(rs+st+rt)+10368(r+s+t)-23328]x^{18}y^{18}(D_{x}^{2}+D_{y}^{2}-2D_{x}D_{y})(M(\mathrm{GCR};x,y)){|}_{x=y=1}=96x^{4}y^{6}+[500(r+s+t)-3000]x^{4}y^{9}+[1296(rs+st+rt)-5184(r+s+t)+1552]x^{4}y^{13}+[2352rst-4704(rs+st+rt)+9408(r+s+t)-18816]x^{4}y^{18}+216x^{6}y^{9}+[128(r+s+t)-768]x^{9}y^{13}+[50(rs+st+rt)-200(r+s+t)+600]x^{13}y^{18}(D_{x}^{2}+D_{y}^{2}-2D_{x}D_{y})(M(\mathrm{GCR};x,y)){|}_{x=y=1}=(96x^{4}y^{6}+[500(r+s+t)-3000]x^{4}y^{9}+[1296(rs+st+rt)-5184(r+s+t)+1552]x^{4}y^{13}+[2352rst-4704(rs+st+rt)+9408(r+s+t)-18816]x^{4}y^{18}+216x^{6}y^{9}+[128(r+s+t)-768]x^{9}y^{13}+[50(rs+st+rt)-200(r+s+t)+600]x^{13}y^{18}){|}_{x=y=1}$$

After putting limits, we have

σ(GCR)=2352rst−3358(rs+st+rt)+4652(r+s+t)−6120

 □

Theorem 11 *If* GCR *be a graph of gold crystal, then the Second Modified Zagreb Index for* M *-Polynomial of* GCR(x,y) *is*

M2m(GCR)=191108rst−82354756(rs+st+rt)+8313689(r+s+t)+501521

Proof In the view of Table 2, applying integral operator $I_{x}$ on Equation (15)

$$\left(I_{x}I_{y})(M(\mathrm{GCR}:x,y))=I_{x}[I_{y}(M(\mathrm{GCR}:x,y)]=I_{x}[4x^{4}y^{6}+[\frac{20}{9}(r+s+t)-\frac{120}{9}]x^{4}y^{9}+[\frac{16}{13}(rs+st+rt)-\frac{64}{13}(r+s+t)+\frac{192}{13}]x^{4}y^{13}+[\frac{2}{3}rst-\frac{4}{3}(rs+st+rt)+\frac{8}{3}(r+s+t)-\frac{16}{3}]x^{4}y^{18}+\frac{24}{9}x^{6}y^{9}+[\frac{4}{9}(r+s+t)-4]x^{9}y^{9}+[\frac{8}{13}(r+s+t)-\frac{48}{13}]x^{9}y^{13}+[\frac{4}{13}(rs+st+rt)-\frac{20}{13}(r+s+t)+\frac{72}{13}]x^{13}y^{13}+[\frac{1}{9}(rs+st+rt)-\frac{4}{9}(r+s+t)+\frac{4}{3}]x^{13}y^{18}+[\frac{1}{6}rst-\frac{7}{18}(rs+st+rt)+\frac{8}{9}(r+s+t)-2]x^{18}y^{18}\right]$$

After simplification, we get

$$(I_{x}I_{y})(M(G:x,y))=x^{4}y^{6}+[\frac{20}{36}(r+s+t)-\frac{120}{36}]x^{4}y^{9}+[\frac{16}{52}(rs+st+rt)-\frac{64}{52}(r+s+t)+\frac{192}{52}]x^{4}y^{13}+[\frac{1}{6}rst-\frac{1}{3}(rs+st+rt)+\frac{2}{3}(r+s+t)-\frac{4}{3}]x^{4}y^{18}+\frac{24}{54}x^{6}y^{9}+[\frac{4}{81}(r+s+t)-\frac{4}{9}]x^{9}y^{9}+[\frac{8}{117}(r+s+t)-\frac{48}{117}]x^{9}y^{13}+[\frac{4}{169}(rs+st+rt)-\frac{20}{169}(r+s+t)+\frac{72}{169}]x^{13}y^{13}+[\frac{1}{117}(rs+st+rt)-\frac{4}{117}(r+s+t)+\frac{4}{36}]x^{13}y^{18}+[\frac{1}{108}rst-\frac{7}{324}(rs+st+rt)+\frac{8}{162}(r+s+t)-\frac{1}{9}]x^{18}y^{18}$$

$$(I_{x}I_{y})(M(\mathrm{GCR}:x,y)){|}_{x=y=1}=(x^{4}y^{6}+[\frac{20}{36}(r+s+t)-\frac{120}{36}]x^{4}y^{9}+[\frac{16}{52}(rs+st+rt)-\frac{64}{52}(r+s+t)+\frac{192}{52}]x^{4}y^{13}+[\frac{1}{6}rst-\frac{1}{3}(rs+st+rt)+\frac{2}{3}(r+s+t)-\frac{4}{3}]x^{4}y^{18}+\frac{24}{54}x^{6}y^{9}+[\frac{4}{81}(r+s+t)-\frac{4}{9}]x^{9}y^{9}+[\frac{8}{117}(r+s+t)-\frac{48}{117}]x^{9}y^{13}+[\frac{4}{169}(rs+st+rt)-\frac{20}{169}(r+s+t)+\frac{72}{169}]x^{13}y^{13}+[\frac{1}{117}(rs+st+rt)-\frac{4}{117}(r+s+t)+\frac{4}{39}]x^{13}y^{18}+[\frac{1}{108}rst-\frac{7}{324}(rs+st+rt)+\frac{8}{162}(r+s+t)-\frac{1}{9})x^{18}y^{18}]{|}_{x=y=1}$$

After putting limits, we have

M2m(GCR)=191108rst−82354756(rs+st+rt)+8313689(r+s+t)+501521

 □

Theorem 12 *If* GCR *be a graph of gold crystal, then the General Randic Index for* M *-Polynomial of* GCR(x,y) *is*

$$R_{\alpha }(\mathrm{GCR})=[12(72^{\alpha })+3(324^{\alpha })]rst+[16(52^{\alpha })-42(72^{\alpha }+4(169^{\alpha }+2(234^{\alpha })-7(324^{\alpha })](rs+st+rt)+[20(36^{\alpha })-64(52^{\alpha })+48(72^{\alpha })+4(81^{\alpha })+8(117^{\alpha })-20(169^{\alpha })-8(234^{\alpha })+16(324^{\alpha })](r+s+t)+24(24^{\alpha })-120(36^{\alpha })+192(52^{\alpha })-96(72^{\alpha })+24(54^{\alpha })-36(81^{\alpha })-48(117^{\alpha })+72(169^{\alpha })+24(234^{\alpha })-36(324^{\alpha })$$

Proof In the view of Table 2 and Theorem 6, we have

$$(D_{x}^{\alpha }D_{y}^{\alpha })(M(\mathrm{GCR};x;y))=D_{x}^{\alpha }D_{y}^{\alpha }(24x^{4}y^{6}+[20(r+s+t)-120]x^{4}y^{9}+[16(rs+st+rt)-64(r+s+t)+192]x^{4}y^{13}+[12rst-24(rs+st+rt)+48(r+s+t)-96]x^{4}y^{18}+24x^{6}y^{9}+[4(r+s+t)-36]x^{9}y^{9}+[8(r+s+t)-48]x^{9}y^{13}+[4(rs+st+rt)-20(r+s+t)+72]x^{13}y^{13}+[2(rs+st+rt)-8(r+s+t)+24]x^{13}y^{18}+[3rst-7(rs+st+rt)+16(r+s+t)-36]x^{18}y^{18})=(D_{x}^{\alpha })({\left(6\right)}^{\alpha }.24x^{4}y^{6}+{\left(9\right)}^{\alpha }[20(r+s+t)-120]x^{4}y^{9}+{\left(13\right)}^{\alpha }[16(rs+st+rt)-64(r+s+t)+192]x^{4}y^{13}+{\left(18\right)}^{\alpha }[12rst-24(rs+st+rt)+48(r+s+t)-96]x^{4}y^{18}+{\left(9\right)}^{\alpha }24x^{6}y^{9}+{\left(9\right)}^{\alpha }[4(r+s+t)-36]x^{9}y^{9}+{\left(13\right)}^{\alpha }[8(r+s+t)-48]x^{9}y^{13}+{\left(13\right)}^{\alpha }[4(rs+st+rt)-20(r+s+t)+72]x^{13}y^{13}+{\left(18\right)}^{\alpha }[2(rs+st+rt)-8(r+s+t)+24]x^{13}y^{18}+{\left(18\right)}^{\alpha }[3rst-7(rs+st+rt)+16(r+s+t)-36]x^{18}y^{18}(D_{x}^{\alpha }D_{y}^{\alpha })(M(\mathrm{GCR};x;y)){|}_{x=y=1}=({\left(24\right)}^{\alpha }.24x^{4}y^{6}+{\left(36\right)}^{\alpha }[20(r+s+t)-120]x^{4}y^{9}+{\left(52\right)}^{\alpha }[16(rs+st+rt)-64(r+s+t)+192]x^{4}y^{13}+{\left(72\right)}^{\alpha }[12rst-24(rs+st+rt)+48(r+s+t)-96]x^{4}y^{18}+{\left(54\right)}^{\alpha }24x^{6}y^{9}+{\left(81\right)}^{\alpha }[4(r+s+t)-36]x^{9}y^{9}+{\left(117\right)}^{\alpha }[8(r+s+t)-48]x^{9}y^{13}+{\left(169\right)}^{\alpha }[4(rs+st+rt)-20(r+s+t)+72]x^{13}y^{13}+{\left(234\right)}^{\alpha }[2(rs+st+rt)-8(r+s+t)+24]x^{13}y^{18}+{\left(324\right)}^{\alpha }[3rst-7(rs+st+rt)+16(r+s+t)-36]x^{18}y^{18}){|}_{x=y=1}$$

After putting limits, we have

$$R_{\alpha }(\mathrm{GCR})=[12(72^{\alpha })+3(324^{\alpha })]rst+[16(52^{\alpha })-24(72^{\alpha })+4(169^{\alpha })+2(234^{\alpha })-7(324^{\alpha })](rs+st+rt)+[20(36^{\alpha })-64(52^{\alpha })+48(72^{\alpha })+4(81^{\alpha })+8(117^{\alpha })-20(169^{\alpha })-8(234^{\alpha })+16(324^{\alpha })](r+s+t)+24(24^{\alpha })-120(36^{\alpha })+192(52^{\alpha })-96(72^{\alpha })+24(54^{\alpha })-36(81^{\alpha })-48(117^{\alpha })+72(169^{\alpha })+24(234^{\alpha })-36(324^{\alpha })$$

 □

Theorem 13 *If* GCR *be a graph of Gold Crystal, then the General Reciprocal Randic Index for* M *-Polynomial of* GCR(x,y) *is*

$$RR_{\alpha }(\mathrm{GCR})=[\frac{12}{{\left(72\right)}^{\alpha }}+\frac{3}{{\left(324\right)}^{\alpha }}]rst+[\frac{16}{{52)}^{\alpha }}-\frac{24}{{\left(72\right)}^{\alpha }}+\frac{4}{{\left(169\right)}^{\alpha })}+\frac{2}{{\left(234\right)}^{\alpha }}-\frac{7}{{\left(324\right)}^{\alpha }}](rs+st+rt)+[\frac{20}{{36)}^{\alpha }}-\frac{64}{{\left(52\right)}^{\alpha }}+\frac{48}{{\left(72\right)}^{\alpha })}+\frac{4}{{\left(81\right)}^{\alpha }}+\frac{8}{{\left(117\right)}^{\alpha }}-\frac{20}{{\left(169\right)}^{\alpha }}-\frac{8}{{\left(234\right)}^{\alpha }}+\frac{16}{{\left(324\right)}^{\alpha }}](r+s+t)+\frac{24}{{\left(24\right)}^{\alpha }}-\frac{120}{{\left(36\right)}^{\alpha }}-\frac{192}{{\left(52\right)}^{\alpha }}-\frac{96}{{\left(72\right)}^{\alpha }}+\frac{24}{{\left(54\right)}^{\alpha }}-\frac{36}{{\left(81\right)}^{\alpha }}-\frac{48}{{\left(117\right)}^{\alpha }}+\frac{72}{{\left(169\right)}^{\alpha }}+\frac{24}{{\left(234\right)}^{\alpha }}-\frac{36}{{\left(324\right)}^{\alpha }}$$

Proof In the view of Table 2 apply the operator on $I_{y}^{\alpha }$ on Equation (12), we have

$$(I_{y}^{\alpha })(M(\mathrm{GCR}:x,y))=\frac{24}{{\left(6\right)}^{\alpha }}x^{4}y^{6}+\frac{1}{{\left(9\right)}^{\alpha }}[20(r+s+t)-120]x^{4}y^{9}+\frac{1}{{\left(13\right)}^{\alpha }}[16(rs+st+rt)-64(r+s+t)+192]x^{4}y^{13}+\frac{1}{{\left(18\right)}^{\alpha }}[12rst-24(rs+st+rt)+48(r+s+t)-96]x^{4}y^{18}+\frac{24}{{\left(9\right)}^{\alpha }}x^{6}y^{9}+\frac{1}{{\left(9\right)}^{\alpha }}[4(r+s+t)-36]x^{9}y^{9}+\frac{1}{{\left(13\right)}^{\alpha }}[8(r+s+t)-48]x^{9}y^{13}+\frac{1}{{\left(13\right)}^{\alpha }}[4(rs+st+rt)-20(r+s+t)+72]x^{13}y^{13}+\frac{1}{{\left(18\right)}^{\alpha }}[2(rs+st+rt)-8(r+s+t)+24]x^{13}y^{18}+\frac{1}{{\left(18\right)}^{\alpha }}[3rst-7(rs+st+rt)+16(r+s+t)-36]x^{18}y^{18}(I_{x}^{\alpha }I_{y}^{\alpha })(M(\mathrm{GCR}:x,y))=\frac{24}{{\left(24\right)}^{\alpha }}x^{4}y^{6}+\frac{1}{{\left(36\right)}^{\alpha }}[20(r+s+t)-120]x^{4}y^{9}+\frac{1}{{\left(52\right)}^{\alpha }}[16(rs+st+rt)-64(r+s+t)+192]x^{4}y^{13}+\frac{1}{{\left(72\right)}^{\alpha }}[12rst-24(rs+st+rt)+48(r+s+t)-96]x^{4}y^{18}+\frac{24}{{\left(54\right)}^{\alpha }}x^{6}y^{9}+\frac{1}{{\left(81\right)}^{\alpha }}[4(r+s+t)-36]x^{9}y^{9}+\frac{1}{{\left(117\right)}^{\alpha }}[8(r+s+t)-48]x^{9}y^{13}+\frac{1}{{\left(169\right)}^{\alpha }}[4(rs+st+rt)-20(r+s+t)+72]x^{13}y^{13}+\frac{1}{{\left(234\right)}^{\alpha }}[2(rs+st+rt)-8(r+s+t)+24]x^{13}y^{18}+\frac{1}{{\left(324\right)}^{\alpha }}[3rst-7(rs+st+rt)+16(r+s+t)-36]x^{18}y^{18}(I_{x}^{\alpha }I_{y}^{\alpha })(M(\mathrm{GCR}:x,y)){|}_{x=y=1}=(\frac{24}{{\left(24\right)}^{\alpha }}x^{4}y^{6}+\frac{1}{{\left(36\right)}^{\alpha }}[20(r+s+t)-120]x^{4}y^{9}+\frac{1}{{\left(52\right)}^{\alpha }}[16(rs+st+rt)-64(r+s+t)+192]x^{4}y^{13}+\frac{1}{{\left(72\right)}^{\alpha }}[12rst-24(rs+st+rt)+48(r+s+t)-96]x^{4}y^{18}+\frac{24}{{\left(54\right)}^{\alpha }}x^{6}y^{9}+\frac{1}{{\left(81\right)}^{\alpha }}[4(r+s+t)-36]x^{9}y^{9}+\frac{1}{{\left(117\right)}^{\alpha }}[8(r+s+t)-48]x^{9}y^{13}+\frac{1}{{\left(169\right)}^{\alpha }}[4(rs+st+rt)-20(r+s+t)+72]x^{13}y^{13}+\frac{1}{{\left(234\right)}^{\alpha }}[2(rs+st+rt)-8(r+s+t)+24]x^{13}y^{18}+\frac{1}{{\left(324\right)}^{\alpha }}[3rst-7(rs+st+rt)+16(r+s+t)-36]x^{18}y^{18}){|}_{x=y=1}$$

After putting limits, we have

$$RR_{\alpha }(\mathrm{GCR})=[\frac{12}{{\left(72\right)}^{\alpha }}+\frac{3}{{\left(324\right)}^{\alpha }}]rst+[\frac{16}{{52)}^{\alpha }}-\frac{24}{{\left(72\right)}^{\alpha }}+\frac{4}{{\left(169\right)}^{\alpha })}+\frac{2}{{\left(234\right)}^{\alpha }}-\frac{7}{{\left(324\right)}^{\alpha }}](rs+st+rt)+[\frac{20}{{36)}^{\alpha }}-\frac{64}{{\left(52\right)}^{\alpha }}+\frac{48}{{\left(72\right)}^{\alpha })}+\frac{4}{{\left(81\right)}^{\alpha }}+\frac{8}{{\left(117\right)}^{\alpha }}-\frac{20}{{\left(169\right)}^{\alpha }}-\frac{8}{{\left(234\right)}^{\alpha }}+\frac{16}{{\left(324\right)}^{\alpha }}](r+s+t)+\frac{24}{{\left(24\right)}^{\alpha }}-\frac{120}{{\left(36\right)}^{\alpha }}-\frac{192}{{\left(52\right)}^{\alpha }}-\frac{96}{{\left(72\right)}^{\alpha }}+\frac{24}{{\left(54\right)}^{\alpha }}-\frac{36}{{\left(81\right)}^{\alpha }}-\frac{48}{{\left(117\right)}^{\alpha }}+\frac{72}{{\left(169\right)}^{\alpha }}+\frac{24}{{\left(234\right)}^{\alpha }}-\frac{36}{{\left(324\right)}^{\alpha }}$$

 □

Theorem 14 *If* GCR *is a graph of gold crystal, then the Redefined Third Zagreb Index of* GCR(x,y) *is*

$$ReZG_{3}=54000rst-73436(rs+st+rt)+95952(r+s+t)-118776$$

Proof From Table 2, Redefined Third Zagreb Index for M-Polynomial is

$$ReZG_{3}(\mathrm{GCR})=(D_{x}D_{y})(D_{x}+D_{y})(M(\mathrm{GCR};x;y)){|}_{x=y=1}$$

From Theorem 1, we have

$$M(\mathrm{GCR};x,y)=24x^{4}y^{6}+[20(r+s+t)-120]x^{4}y^{9}+[16(rs+st+rt)-64(r+s+t)+192]x^{4}y^{13}+[12rst-24(rs+st+rt)+48(r+s+t)-96]x^{4}y^{18}+24x^{6}y^{9}+[4(r+s+t)-36]x^{9}y^{9}+[8(r+s+t)-48]x^{9}y^{13}+[4(rs+st+rt)-20(r+s+t)+72]x^{13}y^{13}+[2(rs+st+rt)-8(r+s+t)+24]x^{13}y^{18}+[3rst-7(rs+st+rt)+16(r+s+t)-36]x^{18}y^{18}(D_{x}+D_{y})(M(G;x,y))=240x^{4}y^{6}+[260(r+s+t)-1560]x^{4}y^{9}+[272(rs+st+rt)-1088(r+s+t)+3264]x^{4}y^{13}+[264rst-528(rs+st+rt)+1056(r+s+t)-2112]x^{4}y^{18}+360x^{6}y^{9}+[72(r+s+t)-648]x^{9}y^{9}+[176(r+s+t)-1056]x^{9}y^{13}+[104(rs+st+rt)-520(r+s+t)+1872]x^{13}y^{13}+[62(rs+st+rt)-248(r+s+t)+744]x^{13}y^{18}+[108rst-252(rs+st+rt)+576(r+s+t)-1296]x^{18}y^{18}$$

$$D_{y}(D_{x}+D_{y})(M(\mathrm{GCR};x;y)=D_{y}(240x^{4}y^{6}+[260(r+s+t)-1560]x^{4}y^{9}+[272(rs+st+rt)-1088(r+s+t)+3264]x^{4}y^{13}+[264rst-528(rs+st+rt)+1056(r+s+t)-2112]x^{4}y^{18}+360x^{6}y^{9}+[72(r+s+t)-648]x^{9}y^{9}+[176(r+s+t)-1056]x^{9}y^{13}+[104(rs+st+rt)-520(r+s+t)+1872]x^{13}y^{13}+[62(rs+st+rt)-248(r+s+t)+744]x^{13}y^{18}+[108rst-252(rs+st+rt)+576(r+s+t)-1296]x^{18}y^{18})D_{y}(D_{x}+D_{y})(M(\mathrm{GCR};x;y)=1440x^{4}y^{6}+[2340(r+s+t)-14040]x^{4}y^{9}+[3536(rs+st+rt)-14144(r+s+t)+42432]x^{4}y^{13}+[4752rst-9504(rs+st+rt)+19008(r+s+t)-38016]x^{4}y^{18}+3240x^{6}y^{9}+[648(r+s+t)-5832]x^{9}y^{9}+[2288(r+s+t)-13728]x^{9}y^{13}+[1352(rs+st+rt)-6760(r+s+t)+24336]x^{13}y^{13}+[1116(rs+st+rt)-4464(r+s+t)+13392]x^{13}y^{18}+[1944rst-4536(rs+st+rt)+10368(r+s+t)-23328]x^{18}y^{18}(D_{x}D_{y})(D_{x}+D_{y})(M(\mathrm{GCR};x;y))=5760x^{4}y^{6}+[9360(r+s+t)-56160]x^{4}y^{9}+[14144(rs+st+rt)-56576(r+s+t)+169728]x^{4}y^{13}+[19008rst-38016(rs+st+rt)+76032(r+s+t)-152064]x^{4}y^{18}+19440x^{6}y^{9}+[5832(r+s+t)-52488]x^{9}y^{9}+[20592(r+s+t)-123552]x^{9}y^{13}+[17576(rs+st+rt)-87880(r+s+t)+316368]x^{13}y^{13}+[14508(rs+st+rt)-58032(r+s+t)+174096]x^{13}y^{18}+[34992rst-81648(rs+st+rt)+186624(r+s+t)-419904]x^{18}y^{18}(D_{x}D_{y})(D_{x}+D_{y})(M(\mathrm{GCR};x;y)){|}_{x=y=1}=(5760x^{4}y^{6}+[9360(r+s+t)-56160]x^{4}y^{9}+[14144(rs+st+rt)-56576(r+s+t)+169728]x^{4}y^{13}+[19008rst-38016(rs+st+rt)+76032(r+s+t)-152064]x^{4}y^{18}+19440x^{6}y^{9}+[5832(r+s+t)-52488]x^{9}y^{9}+[20592(r+s+t)-123552]x^{9}y^{13}+[17576(rs+st+rt)-87880(r+s+t)+316368]x^{13}y^{13}+[14508(rs+st+rt)-58032(r+s+t)+174096]x^{13}y^{18}+[34992rst-81648(rs+st+rt)+186624(r+s+t)-419904]x^{18}y^{18}){|}_{x=y=1}$$

After putting limits, we have

$$ReZG_{3}(\mathrm{GCR})=54000rst-73436(rs+st+rt)+95952(r+s+t)-118776$$

 □

Theorem 15 *If* GCR *is a graph of Gold Crystal, then the Symmetric Division Degree Index of* GCR(x,y) *is*

$$SDD(\mathrm{GCR})=\frac{188}{3}rst-\frac{6809}{117}(rs+st+rt)+\frac{2071}{39}(r+s+t)-\frac{3650}{39}$$

Proof In view of Table 2 along with Equation (15), we have

$$(I_{y})(M(\mathrm{GCR}:x,y))=4x^{4}y^{6}+[\frac{20}{9}(r+s+t)-\frac{120}{9}]x^{4}y^{9}+[\frac{16}{13}(rs+st+rt)-\frac{64}{13}(r+s+t)+\frac{192}{13}]x^{4}y^{13}+[\frac{2}{3}rst-\frac{4}{3}(rs+st+rt)+\frac{8}{3}(r+s+t)-\frac{16}{3}]x^{4}y^{18}+\frac{24}{9}x^{6}y^{9}+[\frac{4}{9}(r+s+t)-4]x^{9}y^{9}+[\frac{8}{13}(r+s+t)-\frac{48}{13}]x^{9}y^{13}+[\frac{4}{13}(rs+st+rt)-\frac{20}{13}(r+s+t)+\frac{72}{13}]x^{13}y^{13}+[\frac{1}{9}(rs+st+rt)-\frac{4}{9}(r+s+t)+\frac{4}{3}]x^{13}y^{18}+[\frac{1}{6}rst-\frac{7}{18}(rs+st+rt)+\frac{8}{9}(r+s+t)-2]x^{18}y^{18}$$

After Applying operator $D_{x}$, we have

$$(D_{x}I_{y})(M(\mathrm{GCR}:x,y))=16x^{4}y^{6}+[\frac{80}{9}(r+s+t)-\frac{480}{9}]x^{4}y^{9}+[\frac{64}{13}(rs+st+rt)-\frac{256}{13}(r+s+t)+\frac{768}{13}]x^{4}y^{13}+[\frac{8}{3}rst-\frac{16}{3}(rs+st+rt)+\frac{32}{3}(r+s+t)-\frac{64}{3}]x^{4}y^{18}+16x^{6}y^{9}+[4(r+s+t)-36]x^{9}y^{9}+[\frac{72}{13}(r+s+t)-\frac{432}{13}]x^{9}y^{13}+[4(rs+st+rt)-20(r+s+t)+72]x^{13}y^{13}+[\frac{13}{9}(rs+st+rt)-\frac{52}{9}(r+s+t)+\frac{52}{3}]x^{13}y^{18}+[3rst-7(rs+st+rt)+16(r+s+t)-36]x^{18}y^{18}$$

From Equation (14), we have

$$D_{y}(M(\mathrm{GCR};x,y))=144x^{4}y^{6}+[180(r+s+t)-1080]x^{4}y^{9}+[208(rs+st+rt)-832(r+s+t)+2496]x^{4}y^{13}+[216rst-432(rs+st+rt)+864(r+s+t)-1728]x^{4}y^{18}+216x^{6}y^{9}+[36(r+s+t)-324]x^{9}y^{9}+[104(r+s+t)-624]x^{9}y^{13}+[52(rs+st+rt)-260(r+s+t)+936]x^{13}y^{13}+[36(rs+st+rt)-144(r+s+t)+432]x^{13}y^{18}+[54rst-126(rs+st+rt)+288(r+s+t)-648]x^{18}y^{18}$$

After operating integral operator $I_{x}$, we have

$$I_{x}D_{y}(M(\mathrm{GCR};x,y))=36x^{4}y^{6}+[45(r+s+t)-270]x^{4}y^{9}+[52(rs+st+rt)-208(r+s+t)+624]x^{4}y^{13}+[54rst-108(rs+st+rt)+216(r+s+t)-432]x^{4}y^{18}+36x^{6}y^{9}+[4(r+s+t)-36]x^{9}y^{9}+[\frac{104}{9}(r+s+t)-\frac{208}{3}]x^{9}y^{13}+[4(rs+st+rt)-20(r+s+t)+72]x^{13}y^{13}+[\frac{36}{13}(rs+st+rt)-\frac{144}{13}(r+s+t)+\frac{432}{13}]x^{13}y^{18}+[3rst-7(rs+st+rt)+16(r+s+t)-36]x^{18}y^{18}(D_{x}I_{y}+I_{x}D_{y})(M(\mathrm{GCR};x,y))=52x^{4}y^{6}+[\frac{485}{9}(r+s+t)-\frac{970}{3}]x^{4}y^{9}+[\frac{740}{13}(rs+st+rt)-\frac{2960}{13}(r+s+t)+\frac{8880}{13}]x^{4}y^{13}+[\frac{170}{3}rst-\frac{340}{3}(rs+st+rt)+\frac{680}{3}(r+s+t)-\frac{1360}{3}]x^{4}y^{18}+52x^{6}y^{9}+[8(r+s+t)-72]x^{9}y^{9}+[\frac{2000}{117}(r+s+t)-\frac{4000}{39}]x^{9}y^{13}+[8(rs+st+rt)-40(r+s+t)+144]x^{13}y^{13}+[\frac{493}{117}(rs+st+rt)-\frac{1972}{117}(r+s+t)+\frac{1972}{39}]x^{13}y^{18}+[6rst-14(rs+st+rt)+32(r+s+t)-72]x^{18}y^{18}(D_{x}I_{y}+I_{x}D_{y})(M(\mathrm{GCR};x,y)){|}_{x=y=1}=(52x^{4}y^{6}+[\frac{485}{9}(r+s+t)-\frac{970}{3}]x^{4}y^{9}+[\frac{740}{13}(rs+st+rt)-\frac{2960}{13}(r+s+t)+\frac{8880}{13}]x^{4}y^{13}+[\frac{170}{3}rst-\frac{340}{3}(rs+st+rt)+\frac{680}{3}(r+s+t)-\frac{1360}{3}]x^{4}y^{18}+52x^{6}y^{9}+[8(r+s+t)-72]x^{9}y^{9}+[\frac{2000}{117}(r+s+t)-\frac{4000}{39}]x^{9}y^{13}+[8(rs+st+rt)-40(r+s+t)+144]x^{13}y^{13}+[\frac{493}{117}(rs+st+rt)-\frac{1972}{117}(r+s+t)+\frac{1972}{39}]x^{13}y^{18}+[6rst-14(rs+st+rt)+32(r+s+t)-72]x^{18}y^{18}){|}_{x=y=1}$$

$$SDD(\mathrm{GCR})=\frac{188}{3}rst-\frac{6809}{117}(rs+st+rt)+\frac{2071}{39}(r+s+t)-\frac{3650}{39}$$

 □

Theorem 16 *If* GCR *be a graph of Gold Crystal, then the Harmonic Index for* M *-Polynomial of* GCR(x,y) *is*

$$H(\mathrm{GCR})=\frac{83}{66}rst-\frac{341335}{1356498}(rs+st+rt)-\frac{18728}{226083}(r+s+t)+\frac{39698}{2431}$$

Proof From Table 2, Harmonic Index for M-Polynomial is

$$H(\mathrm{GCR})=2I_{x}J(M(\mathrm{GCR};x;y)){|}_{x=1}$$

From Theorem 1, we have

$$M(\mathrm{GCR};x,y)=24x^{4}y^{6}+[20(r+s+t)-120]x^{4}y^{9}+[16(rs+st+rt)-64(r+s+t)+192]x^{4}y^{13}+[12rst-24(rs+st+rt)+48(r+s+t)-96]x^{4}y^{18}+24x^{6}y^{9}+[4(r+s+t)-36]x^{9}y^{9}+[8(r+s+t)-48]x^{9}y^{13}+[4(rs+st+rt)-20(r+s+t)+72]x^{13}y^{13}+[2(rs+st+rt)-8(r+s+t)+24]x^{13}y^{18}+[3rst-7(rs+st+rt)+16(r+s+t)-36]x^{18}y^{18}$$

Applying J(f(x,y))=f(x,x) on above equation, we have

$$JM(\mathrm{GCR};x;y)=24x^{10}+[20(r+s+t)-120]x^{13}+24x^{15}+[16(rs+st+rt)-64(r+s+t)+192]x^{17}+[4(r+s+t)-36]x^{18}+[12rst-24(rs+st+rt)+56(r+s+t)-144]x^{22}+[4(rs+st+rt)-20(r+s+t)+72]x^{26}+[2(rs+st+rt)-8(r+s+t)+24]x^{31}+[3rst-7(rs+st+rt)+16(r+s+t)-36]x^{36}$$

After operating integral operator $I_{x}$ (10), we have

$$I_{x}JM(\mathrm{GCR};x;y)=\frac{12}{5}x^{10}+[\frac{20}{13}(r+s+t)-\frac{120}{13}]x^{13}+\frac{24}{15}x^{15}+[\frac{16}{17}(rs+st+rt)-\frac{64}{17}(r+s+t)+\frac{192}{17}]x^{17}+[\frac{2}{9}(r+s+t)-2]x^{18}+[\frac{6}{11}rst-\frac{12}{11}(rs+st+rt)+\frac{28}{11}(r+s+t)-\frac{72}{11}]x^{22}+[\frac{2}{13}(rs+st+rt)-\frac{10}{13}(r+s+t)+\frac{36}{13}]x^{26}+[\frac{2}{31}(rs+st+rt)-\frac{8}{31}(r+s+t)+\frac{24}{31}]x^{31}+[\frac{1}{12}rst-\frac{7}{36}(rs+st+rt)+\frac{4}{9}(r+s+t)-1]x^{36}$$

$$2I_{x}JM(\mathrm{GCR};x;y)=\frac{24}{5}x^{10}+[\frac{40}{13}(r+s+t)-\frac{240}{13}]x^{13}+\frac{48}{15}x^{15}+[\frac{32}{17}(rs+st+rt)-\frac{128}{17}(r+s+t)+\frac{384}{17}]x^{17}+[\frac{4}{9}(r+s+t)-4]x^{18}+[\frac{12}{11}rst-\frac{24}{11}(rs+st+rt)+\frac{56}{11}(r+s+t)-\frac{144}{11}]x^{22}+[\frac{4}{13}(rs+st+rt)-\frac{20}{13}(r+s+t)+\frac{72}{13}]x^{26}+[\frac{4}{31}(rs+st+rt)-\frac{16}{31}(r+s+t)+\frac{48}{31}]x^{31}+[\frac{1}{6}rst-\frac{14}{36}(rs+st+rt)+\frac{8}{9}(r+s+t)-2]x^{36}\;2I_{x}JM(\mathrm{GCR};x;y){|}_{x=1}=(\frac{24}{5}x^{10}+[\frac{40}{13}(r+s+t)-\frac{240}{13}]x^{13}+\frac{48}{15}x^{15}+[\frac{32}{17}(rs+st+rt)-\frac{128}{17}(r+s+t)+\frac{384}{17}]x^{17}+[\frac{4}{9}(r+s+t)-4]x^{18}+[\frac{12}{11}rst-\frac{24}{11}(rs+st+rt)+\frac{56}{11}(r+s+t)-\frac{144}{11}]x^{22}+[\frac{4}{13}(rs+st+rt)-\frac{20}{13}(r+s+t)+\frac{72}{13}]x^{26}+[\frac{4}{31}(rs+st+rt)-\frac{16}{31}(r+s+t)+\frac{48}{31}]x^{31}+[\frac{1}{6}rst-\frac{14}{36}(rs+st+rt)+\frac{8}{9}(r+s+t)-2]x^{36}){|}_{x=1}$$

$$H(\mathrm{GCR})=\frac{83}{66}rst-\frac{341335}{1356498}(rs+st+rt)-\frac{18728}{226083}(r+s+t)+\frac{39698}{2431}$$

 □

Theorem 17 *If* GCR *be a graph of Gold Crystal, then the Inverse Sum Index for* M *-Polynomial of* GCR(x,y) *is*

$$I(\mathrm{GCR})=\frac{729}{11}rst-\frac{298589}{5797}(rs+st+rt)-\frac{148419}{4808}(r+s+t)-\frac{264573}{36209}$$

Proof In view of Table 2 and Theorem 5, we have

$$D_{x}D_{y}(M(\mathrm{GCR};x;y))=576x^{4}y^{6}+[720(r+s+t)-4320]x^{4}y^{9}+[832(rs+st+rt)-3328(r+s+t)+9984]x^{4}y^{13}+[864rst-1728(rs+st+rt)+3456(r+s+t)-6912]x^{4}y^{18}+1296x^{6}y^{9}+[324(r+s+t)-2916]x^{9}y^{9}+[936(r+s+t)-5616]x^{9}y^{13}+[676(rs+st+rt)-3380(r+s+t)+12168]x^{13}y^{13}+[468(rs+st+rt)-1872(r+s+t)+5616]x^{13}y^{18}+[972rst-2268(rs+st+rt)+5184(r+s+t)-11664]x^{18}y^{18}$$

Apply J(f(x,y))=f(x,x) on above equation, we have

$$JD_{x}D_{y}(M(\mathrm{GCR};x;y))=576x^{10}+[720(r+s+t)-4320]x^{13}+1296x^{15}+[832(rs+st+rt)-3328(r+s+t)+9984]x^{17}+[324(r+s+t)-2916]x^{18}+[864rst-1728(rs+st+rt)+4392(r+s+t)-12528]x^{22}+[676(rs+st+rt)-3380(r+s+t)+12168]x^{26}+[468(rs+st+rt)-1872(r+s+t)+5616]x^{31}+[972rst-2268(rs+st+rt)+5184(r+s+t)-11664]x^{36}$$

After operating integral operator $I_{x}$ (10), we have

$$I_{x}JD_{x}D_{y}(M(\mathrm{GCR};x;y))=\frac{288}{5}x^{10}+[\frac{720}{13}(r+s+t)-\frac{4320}{13}]x^{13}+\frac{432}{5}x^{15}+[\frac{832}{17}(rs+st+rt)-\frac{3328}{17}(r+s+t)+\frac{9984}{17}]x^{17}+[18(r+s+t)-162]x^{18}+[\frac{432}{11}rst-\frac{864}{11}(rs+st+rt)+\frac{2196}{11}(r+s+t)-\frac{6264}{11}]x^{22}+[26(rs+st+rt)-130(r+s+t)+468]x^{26}+[\frac{468}{31}(rs+st+rt)-\frac{1872}{31}(r+s+t)+\frac{5616}{31}]x^{31}+[27rst-63(rs+st+rt)+144(r+s+t)-324]x^{36}\;I_{x}JD_{x}D_{y}(M(\mathrm{GCR};x;y)){|}_{x=1}=(\frac{288}{5}x^{10}+[\frac{720}{13}(r+s+t)-\frac{4320}{13}]x^{13}+\frac{432}{5}x^{15}+[\frac{832}{17}(rs+st+rt)-\frac{3328}{17}(r+s+t)+\frac{9984}{17}]x^{17}+[18(r+s+t)-162]x^{18}+[\frac{432}{11}rst-\frac{864}{11}(rs+st+rt)+\frac{2196}{11}(r+s+t)-\frac{6264}{11}]x^{22}+[26(rs+st+rt)-130(r+s+t)+468]x^{26}+[\frac{468}{31}(rs+st+rt)-\frac{1872}{31}(r+s+t)+\frac{5616}{31}]x^{31}+[27rst-63(rs+st+rt)+144(r+s+t)-324]x^{36}){|}_{x=1}$$

$$I(\mathrm{GCR})=\frac{729}{11}rst-\frac{298589}{5797}(rs+st+rt)-\frac{148419}{4808}(r+s+t)-\frac{264573}{36209}$$

 □

The article "Computation of differential and integral operators using ℳ-polynomials of gold crystal" was retracted in 2025. Reasons: plagiarism; unreliable results or conclusions; concerns about the peer review; concerns about the citations.

## 4 Numerical and graphical comparative analysis of computed TIs

The computational values of TIs are presented in Table 3, Table 4, Table 5, we take the same values ranging from 3 to 9 for r, s and t for numerical computation purposes. We also presented a graphical representation of these computational values in Fig. 2. It is observed as values of r, s and t increased the TIs values also increased gradually.

**Table 3:** Numerical values of $M_{1}\left(\mathrm{GCR}\right)$, $M_{2}\left(\mathrm{GCR}\right)$, HM(GCR) and σ(GCR).

(r,s,t)	$M_{1}\left(\mathrm{GCR}\right)$	$M_{2}\left(\mathrm{GCR}\right)$	HM(GCR)	σ(GCR)
(3,3,3)	3174	11604	55002	8586
(4,4,4)	10608	43236	211992	39048
(5,5,5)	24918	106812	533058	105810
(6,6,6)	48336	213348	1076376	222984
(7,7,7)	83094	373860	1900122	404682
(8,8,8)	131424	599364	3062472	665016
(9,9,9)	195558	9008762	4621602	1018098

**Table 4:** Computational values of M2m(GCR), $R_{\alpha }\left(\mathrm{GCR}\right)$, $RR_{\alpha }\left(\mathrm{GCR}\right)$, $ReZG_{3}\left(\mathrm{GCR}\right)$.

(r,s,t)	M2m(GCR)	$R_{\alpha }\left(\mathrm{GCR}\right)$	$RR_{\alpha }\left(\mathrm{GCR}\right)$	$ReZG_{3}\left(\mathrm{GCR}\right)$
(3,3,3)	0.14462	198484.511061	28.846615	220020
(4,4,4)	0.48165	363616.577195	75.956968	963720
(5,5,5)	1.14005	579954.192927	157.647974	2562804
(6,6,6)	2.222709	848432.298514	283.404914	5341272
(7,7,7)	3.832514	1169985.834216	462.713069	9623124
(8,8,8)	6.072354	1545549.740291	705.057721	15732360
(9,9,9)	9.045117	1976058.956999	1019.924151	23992980

The article "Computation of differential and integral operators using ℳ-polynomials of gold crystal" was retracted in 2025. Reasons: plagiarism; unreliable results or conclusions; concerns about the peer review; concerns about the citations.

**Table 5:** Computational values of SDD(GCR), H(GCR), I(GCR).

(r,s,t)	SDD(GCR)	H(GCR)	I(GCR)
(3,3,3)	505.025641	42.744921	113.531614
(4,4,4)	1760.871795	83.742493	1391.357413
(5,5,5)	4171.538462	153.412105	3950.683643
(6,6,6)	8113.025641	259.299213	8189.146667
(7,7,7)	13961.333333	408.949271	14504.38285
(8,8,8)	22092.461538	609.907733	23294.028556
(9,9,9)	32882.410256	869.720054	34955.720147

**Figure 2:** Graphical comparison of numerical values of TIs.

## Conclusion

In this study, we have computed the M-Polynomial for the structure of Gold crystal

$$M(\mathrm{GCR};x,y)=24x^{4}y^{6}+[20(r+s+t)-120]x^{4}y^{9}+[16(rs+st+rt)-64(r+s+t)+192]x^{4}y^{13}+[12rst-24(rs+st+rt)+48(r+s+t)-96]x^{4}y^{18}+24x^{6}y^{9}+[4(r+s+t)-36]x^{9}y^{9}+[8(r+s+t)-48]x^{9}y^{13}+[4(rs+st+rt)-20(r+s+t)+72]x^{13}y^{13}+[2(rs+st+rt)-8(r+s+t)+24]x^{13}y^{18}+[3rst-7(rs+st+rt)+16(r+s+t)-36]x^{18}y^{18}$$

and the differential operators for GCR(x,y) are

$$D_{x}(M(\mathrm{GCR};x,y))=96x^{4}y^{6}+[80(r+s+t)-480]x^{4}y^{9}+[64(rs+st+rt)-256(r+s+t)+768]x^{4}y^{13}+[48rst-96(rs+st+rt)+192(r+s+t)-384]x^{4}y^{18}+144x^{6}y^{9}+[36(r+s+t)-324]x^{9}y^{9}+[72(r+s+t)-432]x^{9}y^{13}+[52(rs+st+rt)-260(r+s+t)+936]x^{13}y^{13}+[26(rs+st+rt)-104(r+s+t)+312]x^{13}y^{18}+[54rst-126(rs+st+rt)+288(r+s+t)-648]x^{18}y^{18}$$

and

$$D_{y}(M(\mathrm{GCR};x,y))=144x^{4}y^{6}+[180(r+s+t)-1080]x^{4}y^{9}+[208(rs+st+rt)-832(r+s+t)+2496]x^{4}y^{13}+[216rst-432(rs+st+rt)+864(r+s+t)-1728]x^{4}y^{18}+216x^{6}y^{9}+[36(r+s+t)-324]x^{9}y^{9}+[104(r+s+t)-624]x^{9}y^{13}+[52(rs+st+rt)-260(r+s+t)+936]x^{13}y^{13}+[36(rs+st+rt)-144(r+s+t)+432]x^{13}y^{18}+[54rst-126(rs+st+rt)+288(r+s+t)-648]x^{18}y^{18}$$

The integral operators for GCR(x,y) are

$$I_{x}(M(\mathrm{GCR};x,y)))=6x^{4}y^{6}+[5(r+s+t)-30]x^{4}y^{9}+[4(rs+st+rt)-16(r+s+t)+48]x^{4}y^{13}+[3rst-6(rs+st+rt)+12(r+s+t)-24]x^{4}y^{18}+4x^{6}y^{9}+[\frac{4}{9}(r+s+t)-4]x^{9}y^{9}+[\frac{8}{9}(r+s+t)-\frac{48}{9}]x^{9}y^{13}+[\frac{4}{13}(rs+st+rt)-\frac{20}{13}(r+s+t)+\frac{72}{13}]x^{13}y^{13}+[\frac{2}{13}(rs+st+rt)-\frac{8}{13}(r+s+t)+\frac{24}{13}]x^{13}y^{18}+[\frac{1}{6}rst-\frac{7}{18}(rs+st+rt)+\frac{8}{9}(r+s+t)-2]x^{18}y^{18}$$

and

$$I_{y}(M(\mathrm{GCR};x,y)))=4x^{4}y^{6}+[\frac{20}{9}(r+s+t)-\frac{120}{9}]x^{4}y^{9}+[\frac{16}{13}(rs+st+rt)-\frac{64}{13}(r+s+t)+\frac{192}{13}]x^{4}y^{13}+[\frac{2}{3}rst-\frac{4}{3}(rs+st+rt)+\frac{8}{3}(r+s+t)-\frac{16}{3}]x^{4}y^{18}+\frac{24}{9}x^{6}y^{9}+[\frac{4}{9}(r+s+t)-4]x^{9}y^{9}+[\frac{8}{13}(r+s+t)-\frac{48}{13}]x^{9}y^{13}+[\frac{4}{13}(rs+st+rt)-\frac{20}{13}(r+s+t)+\frac{72}{13}]x^{13}y^{13}+[\frac{1}{9}(rs+st+rt)-\frac{4}{9}(r+s+t)+\frac{4}{3}]x^{13}y^{18}+[\frac{1}{6}rst-\frac{7}{18}(rs+st+rt)+\frac{8}{9}(r+s+t)-2]x^{18}y^{18}$$

We also computed the eleven topological indices of GCR by employing the M-Polynomial, the differential and integral operators. The numerical and graphical comparison of these indices is also employed. These results shall also attract the researchers to explore new results for other molecular structures by using this methodology.

The article "Computation of differential and integral operators using ℳ-polynomials of gold crystal" was retracted in 2025. Reasons: plagiarism; unreliable results or conclusions; concerns about the peer review; concerns about the citations.

## Funding

No funds, grants, or other support were received.

## CRediT authorship contribution statement

**Abdul Rauf Khan:** Writing – review & editing, Validation, Investigation, Conceptualization, Data curation, Formal analysis, Methodology, Resources, Software, Visualization. **Saad Amin Bhatti:** Visualization, Software, Resources, Methodology. **Muhammad Imran:** Software, Funding acquisition, Formal analysis, Data curation. **Ferdous M.O. Tawfiq:** Writing – review & editing, Writing – original draft, Validation, Formal analysis, Data curation, Conceptualization, Investigation, Methodology. **Murat Cancan:** Writing – review & editing, Visualization, Software, Methodology, Investigation. **Shahid Hussain:** Writing – review & editing, Validation, Resources, Methodology.

## Declaration of Competing Interest

The authors declare that they have no known competing financial interests or personal relationships that could have appeared to influence the work reported in this paper.

## Data Availability

No data was used for the research described in the article.
